# Transparent Meta-Analysis of Prospective Memory and Aging

**DOI:** 10.1371/journal.pone.0001568

**Published:** 2008-02-20

**Authors:** Bob Uttl

**Affiliations:** Red Deer College, Red Deer, Alberta, Canada; University of Southern California, United States of America

## Abstract

Prospective memory (ProM) refers to our ability to become aware of a previously formed plan at the right time and place. After two decades of research on prospective memory and aging, narrative reviews and summaries have arrived at widely different conclusions. One view is that prospective memory shows large age declines, larger than age declines on retrospective memory (RetM). Another view is that prospective memory is an exception to age declines and remains invariant across the adult lifespan. The present meta-analysis of over twenty years of research settles this controversy. It shows that prospective memory declines with aging and that the magnitude of age decline varies by prospective memory subdomain (vigilance, prospective memory proper, habitual prospective memory) as well as test setting (laboratory, natural). Moreover, this meta-analysis demonstrates that previous claims of no age declines in prospective memory are artifacts of methodological and conceptual issues afflicting prior research including widespread ceiling effects, low statistical power, age confounds, and failure to distinguish between various subdomains of prospective memory (e.g., vigilance and prospective memory proper).

## Introduction

Prospective memory refers to our ability to become aware of a previously formed plan at the right time and place, for example, becoming aware of the plan to buy groceries while passing by a supermarket [1]. While Craik [2], [3] sparked initial interest in age-related changes in prospective memory by theoretical analysis suggesting that age declines in prospective memory would be large, at least as large, or larger than age declines in retrospective memory, Einstein and McDaniel [4] propelled research forward by claiming that ProM is an “exciting exception to typically found age-related decrements in memory” (p. 724).”

More than two decades of research later, the divide between Craik's [2], [3] and Einstein and McDaniel's [4] claims appears to be as deep as ever; narrative reviews and summaries of the effects of aging on prospective memory have arrived at widely different conclusions. While some researchers view the literature as showing no age-related declines in prospective memory, others see the literature as showing “substantial” age-related declines. On one side of this controversy firmly stands Einstein and McDaniel's [4] study purportedly showing that prospective memory ability does not decline with aging. More than a decade later, McDaniel, Einstein, Stout and Morgan [5] summarized 20 years of research with the following: “Although the pattern of age-related effects is mixed, a significant number of studies show little or no age-related decrements in prospective memory performance on this [typical] event-based prospective memory task”. Most recently, McDaniel and Einstein presented data purportedly showing age-invariance with focal prospective cues [6] and argued that this is due to “automatic”, “reflexive”, or “obligatory” retrieval of the plan in response to the appearance of the prospective memory cue [6]–[8]. On the other side of this controversy are authors who conclude that prospective memory shows substantial age-related declines. To illustrate, Craik and Bialystok [9] consider age-related decrements in prospective memory “established”(see also [10]–[12]).

The vastly different interpretations of previous research on prospective memory and aging suggest that a systematic objective quantitative review of the last 25 years is needed to determine the status of the field and provide guidance for the future. Are age declines in prospective memory as large or larger than in retrospective memory as suggested by Craik [2], [3]or is prospective memory “an exciting exception to typically found age-related decrements in memory”? Are there a substantial number of studies showing no decline? And if so, what are their characteristics? What factors are correlated with the size of age declines observed in different studies? What are the reasons for this profound disagreement about the interpretation of two decades of research on prospective memory and aging?

One of the first meta-analyses of prospective memory research findings by Birt [13] concluded that prospective memory showed robust declines on laboratory prospective memory tasks but improvements on naturalistic prospective memory tasks. A more recent meta-analysis by Henry, MacLeod, Phillips, and Crawford [14] confirmed Birt's [13] findings and made two additional claims. First, Henry et al. concluded that age declines were smaller for prospective memory tasks supported by relatively automatic processes and larger for prospective memory tasks supported by relatively effortful processes. Second, Henry et al. concluded that age declines in prospective memory were smaller than age declines in retrospective memory, contrary to Craik's [2], [3] proposal. Most recently, Uttl [15], [16] reported that many studies of prospective memory suffer from severe ceiling effects, low statistical power, poor reliability, and poor validity. Moreover, he found that the best predictor of the size of age declines in one subdomain of prospective memory (event-cued) was the researcher's ability to avoid ceiling effects–performance on easy prospective memory tests showed no age declines because both age groups achieved perfect or nearly perfect scores and performance on more difficult tests showed larger age declines. In turn, Uttl's [15], [16] findings suggest that the results of Henry et al.'s meta-analysis may be misleading as they did not take into account the prevalent ceiling effects that serve to artificially reduce the effect sizes reported in their meta-analysis.

As an illustrative example, Figure 1 demonstrates the undesirable effects of ceiling-limited data on the magnitude of age declines on low versus high demand prospective memory tasks included in Henry et al.'s [14] meta-analysis. Henry et al. [14] reported an average effect size for low (*r* = −.14 or *d* = −0.28) versus high (*r* = −.40 or *d* = −0.87) demand conditions, together with the required *k*s, *Q*s, and *p*s, and concluded that age declines are much smaller in low demand than in high demand prospective memory tasks. However, an evaluation of the quality of included studies and quality of primary data reveals that this conclusion is unwarranted. Figure 1a shows a box plot of individual study effect sizes obtained from Henry et al. [14]; the figure reveals, consistent with Henry et al.'s conclusions, that low demand conditions are associated with smaller effect sizes than high demand conditions. It also shows that there appears to be an outlier in the low demand condition, suggesting possible heterogeneity. Figure 1b and 1c show forest plots of individual effect sizes for low versus high demand conditions; they are more informative and transparent as they reveal individual effect sizes for each age contrast with the size of the effect size marker related to the size of the study. Although the number of the studies is small, the data in Figure 1b suggest heterogeneity, that is widely varying effect sizes, and the data in Figure 1c suggest that the magnitude of age declines reported by Cherry and her colleagues [17] are smaller than those reported by other investigators. A follow-up examination of the method section reveals that Cherry and her colleagues confounded age with intelligence by comparing very intelligent older adults with not so intelligent younger adults, and thus, the smaller age declines observed in this set of studies may be attributable to this intelligence confound.

**Figure 1:** The impact of abstraction in presenting results of meta-analysis using the Henry et al. [14] meta-analysis of low versus high demand ProM as an example. Figure 1a shows a box plot of individual study effect sizes obtained by Henry et al. including the effect size *d* indices; the figure suggests, consistent with Henry et al.'s conclusion, that the low demand conditions (in blue) are associated with smaller effect sizes than the high demand conditions (in red). Figures 1b and 1c show forest plots of individual effect sizes for low and high demand conditions, respectively, with the size of the effect size marker indicating the size of the study and the horizontal line indicating the confidence interval for the size effect. Figure 1b suggests heterogeneity whereas Figure 1c suggests that the effect sizes reported by Cherry and her colleagues are smaller than the effect sizes obtained by other investigators. Figure 1d shows a plot of actual primary data with the x-axis showing performance of older adults (mean success proportion) and the y-axis showing performance of younger adults (mean success proportion) with low versus high demand conditions indicated by blue circles and red squares, respectively, and the size of the markers indicating the sample size of the study. The dashed markers identify age contrasts that are limited by severe ceiling effects, that is, where performance of at least one of the groups is over 0.90, and the size of age declines is severely underestimated. Figure 1d indicates that the summary effect sizes in Figure 1a, as well as individual effect sizes in the forest plots of Figure 1b and 1c, substantially underestimate the true effect size simply due to an artificial limit on the effect size due to severe ceiling effects. The dashed markers in Figure 1e identify studies that confounded age with experimental design (i.e., ongoing task was easier for older versus younger adults), and therefore, artificially reduced the size of observed age declines. Figure 1f shows that when ceiling limited and age-confounded age contrasts are removed from the Henry et al. [14] meta-analysis, we are left with only two low- and two high-demand age contrasts (see Figure 1f) arising from two experiments from a single article by Einstein, Smith, McDaniel, and Shaw [20]. Unfortunately, careful reading of the method section reveals that Einstein et al. [20] did not include any delay between ProM instructions and task performance, and thus, performance reflects vigilance rather than ProM proper.

Looking at the same data in another way, Figure 1d shows a plot of actual primary data with the x-axis showing performance of older adults (mean success proportion) and the y-axis showing performance of younger adults (mean success proportion) with low versus high demand conditions indicated by circles and squares, respectively, and the size of the markers indicating the sample size of the study. The dashed markers identify age contrasts that are limited by severe ceiling effects, that is, where performance of at least one group is over .90, and the size of age declines is underestimated [17]–[19]. To illustrate, Henry et al. [14] reported an effect size *d* = 0 for the low demand condition of Kidder et al. [18] but both young and older adults obtained accuracy scores of 0.98 in this condition, suggesting that the test was too easy (see circles in the top right corner of Figure 1d). The left panel of Figure 2 shows raw non-standardized performance by younger and older adults in Kidder et al. study and highlight that severe ceiling effects in the low demand condition are solely responsible for *d* = 0. Similarly, the right panel of Figure 2 reveals a similar ceiling effect problem with another study included in Henry et al. analysis. Accordingly, the summary effect sizes in Figure 1a, as well as individual effect sizes in the forest plots of Figure 1b, substantially underestimate the true effect size due to artificial limits imposed by ceiling effects. Moreover, these ceiling effect artifacts cannot be detected by plotting individual effect sizes and they are undetectable by graphs such as stem-and-leaf, box, or forest plots.

**Figure 2:** The left panel shows raw non-standardized performance by younger and older adults in low and high demand conditions in Kidder et al. [18], one of the studies included in Henry et al. [14] meta-analysis. The figure makes it obvious that performance in “low” demand conditions was so high as to be nearly perfect whereas performance in “high” demand conditions was generally lower. Ignoring the obvious ceiling effects, Henry et al. reported an effect size of *r* = 0 for the low demand condition and an effect size of *r* = −0.47 for the high demand condition (see Appendix A, Henry et al. [14]). Similarly, the right panel reveals a similar ceiling effect problem with the study by Park et al. [19] included in this same meta-analysis.

In Figure 1e, the dashed markers identify studies that confounded age with experimental design (i.e., ongoing task was easier for older versus younger adults) [8], [17], and therefore, should not have been included in the meta-analysis of age differences or should have been analyzed separately. When ceiling limited and age-confounded age contrasts are removed from this meta-analysis, we are left with only two low- and two high-demand age contrasts (see Figure 1f) arising from two experiments from a single article by Einstein, Smith, McDaniel, and Shaw [20]. Moreover, a close inspection of Einstein et al.'s method section reveals that these two experiments did not include a delay between the prospective memory instructions and the start of the ongoing task, a condition considered necessary for the task to allow assessment of prospective memory rather than vigilance [1], [7], [21], [22]. This simple example of a recently published and often quoted meta-analysis shows that summary effect sizes and associated confidence intervals may be highly misleading when primary data suffer from fundamental problems such as restricted range due to ceiling or floor effects. Thus, a new quantitative review of prospective memory that takes these issues into account (e.g., restricted range, low reliability, design confounds, etc.) is necessary to settle the 20 year old controversy about age declines in prospective memory.

Accordingly, this article presents a new meta-analysis of the accumulated research on prospective memory and aging to determine the extent of age declines in prospective memory, while taking into account methodological characteristics of the primary studies. Craik [2], [3] suggested that age declines on prospective memory are larger than on free recall (*d* = 1.01, Spencer & Raz [23], .*d* = 0.97, La Voie & Light [24]). If this view is correct, then we should observe age declines corresponding to *d* = 1.0 or more. However, if prospective memory is spared by aging, or spared by aging under some circumstances as argued by McDaniel, Einstein, and their colleagues, we should find no age declines in methodologically sound studies unaffected by ceiling effects and design confounds. To ensure the transparency, informativeness, and robustness of the present meta-analysis, the data are analyzed using robust count methods, graphical methods and modeling of primary data as well as by more traditional methods.

The present meta-analysis also addresses several important questions and controversies that have not been addressed or have been addressed only partially in the previous meta-analyses. First, if prospective memory declines with aging, what is the pattern of such declines? Are declines linear across the adult life span or are they curvilinear with accelerated declines after about 50–60 years of age? Second, do age declines vary across prospective memory subdomain (i.e., vigilance, prospective memory proper, habitual prospective memory), cue type (event, time), and experimental setting (laboratory versus naturalistic)? To illustrate, although the previous meta-analyses noted age improvements in naturalistic settings and age declines or no changes in laboratory settings, if studies in laboratory versus naturalistic settings examined different aspects of prospective memory (e.g., event-cued versus time-cued prospective memory) their conclusions may be unwarranted to the extent to which age effects vary across prospective memory subdomain and cue type. Naturally, this possibility leads to the third question: What aspects of prospective memory have been investigated to date and what aspects remain uninvestigated? The next sections present a review of the necessary concepts and long-standing controversies in the field, beginning with the controversy of how to define prospective memory.

### Prospective memory: What is it?

What is prospective memory? Prospective memory has been variously defined as “remembering to do something in the future” [25], “remembering to do something in the future without being reminded” [26], “timely execution of an intended action at some point in the future” [27], “realization of delayed intentions” [10], “memory for activities to be performed in the future” [4], “remembering to remember” [28], and so on. This sampler of definitions suggests considerable variation in researchers' conception of what prospective memory is; by all of these definitions, prospective memory is required for such diverse tasks as monitoring a kettle, remembering to get groceries en route home from work, returning a library book by the due date, and taking high blood pressure medication every day. Consistent with these definitions, researchers have used performance on a wide variety of tasks as indices of prospective memory. For example, West and Craik [10] required participants to classify briefly presented words according to print color or semantic category (ongoing task) and to press an assigned key whenever the prospective memory cue occurred; they then used the proportion of detected cue words as an index of prospective memory. Tombaugh, Grandmaison, and Schmidt [29] required participants to memorize six different prospective memory cue-task pairs, to perform the correct action in response to each prospective memory cue, and used the proportion of correctly performed tasks as an index of prospective memory. Moscovitch [30] required participants to call the experimenter every day for two weeks at the same pre-arranged time. Perhaps not surprisingly, this wide variation in definitions, conceptions, and operationalization of prospective memory, as well as apparent overlap with well-known fields such as studies of vigilance, may appear confusing to a newcomer and has led to severe criticisms of the field [31], [32] and even the suggestion that “the loss of the term of prospective memory would leave us better off, not impoverished” [31]. What then is “prospective memory”? What makes it unique and why should we not simply discard the term?

We [1] have argued elsewhere that one of the distinguishing features of prospective memory, as opposed to retrospective memory, is the recognition of cues as signs of a previously formed plan when the cues appear as part of ongoing thoughts, actions, or situations [1] (see also Craik [2], [3]). To illustrate, when driving by the supermarket en route home, no one alerts us to the relevance of this cue to the previously formed plan (buying groceries) and no one instructs us that the cue signals that now is the time to become aware of the plan, recollect it, and execute it. In contrast, for all retrospective memory tasks, participants are alerted to the presence of the cues (e.g., word stems) and instructed to work with them in a task-relevant manner (e.g., recall all previously studied words that start with the stems [explicit memory] or complete the stems with the first word that comes to mind [implicit memory]). Thus, the unique aspect of prospective memory is bringing a previously formed plan back to consciousness at the right time and place [1], [16], [21], [33] (see also [7]). However, the definitions of prospective memory cited above, experimental tasks purportedly assessing prospective memory, paper abstracts, and papers themselves frequently make no reference to this unique function of prospective memory and do not distinguish between tasks that do versus do not require this unique component of prospective memory. One prospective memory paper uses a task that requires this unique function of prospective memory whereas another prospective memory paper uses a variant of a venerable vigilance task. This situation is confusing, as confusing as purging terms like “short-term/working memory”, “long-term (episodic) memory”, “semantic memory”, and “implicit memory” from our vocabulary in favor of one single non-specific term “retrospective memory” and then arguing about whether there are memory age declines or age improvements in retrospective memory. Indeed, we [1] view the term “prospective memory” as an umbrella term, comprised of several subdomains, just as “retrospective memory” is an umbrella term for short-term memory, episodic long-term memory, semantic memory, etc. (see Table 1).

**Table 1:** The subdomains of retrospective and prospective memory

Retrospective memory	Prospective memory
**Short-term/Working memory**	**Vigilance/monitoring**
Looking up and dialing phone number	Preventing a kettle from boiling over
**Long-term memory**	**ProM proper (ProMP)**
Encoding and recollecting past events	Buying groceries en route home
**Semantic memory**	**Habitual ProM (HproM)**
Knowing facts, things, & procedures	Taking same medication every evening

#### Subdomains of prospective memory

In response to Crowder's [31] and Roediger's [32] criticism, Graf and Uttl [1] delineated the unique function of prospective memory, drew a parallel between subdomains of retrospective memory (short-term, long-term, and semantic memory), and argued for a distinction between different subdomains of prospective memory: prospective memory proper (ProMP), vigilance, and habitual prospective memory (HProM) (see Table 1). Specifically, they argued that the unique function of prospective memory proper (cf. episodic prospective memory [33]) is to bring back to awareness previously formed plans and intentions at the right place and time to allow us to act upon those plans and intentions. A typical situation requiring prospective memory proper is to buy groceries en route home from work as illustrated in Figure 3. We make a plan to buy groceries but then we go about our daily activities and do not maintain the plan in consciousness. The function of prospective memory proper is to bring the plan back to consciousness at the right time and place, when we are approaching the prospective memory cue, a supermarket. To retrieve the content of the plan, which groceries to buy, is the function of retrospective memory.

**Figure 3:** A typical situation requiring ProM proper (prospective memory proper) is to buy groceries en route home from work. We make a plan to buy groceries but then we go about our daily activities and do not maintain the plan in consciousness. The function of prospective memory proper is to bring the plan back to consciousness at the right time and place, when we are approaching the ProM cue, a supermarket.

Vigilance differs from prospective memory proper in that the plan remains in consciousness [1], [21], [33]. To illustrate, an air-traffic controller maintains a plan in consciousness–to issue orders to ensure separation of airplanes–and watches out for occurrences of cues to issue such orders. Although this key distinction between prospective memory proper and vigilance–the requirement to retrieve the plan and bring it back to consciousness–is widely acknowledged, it is rarely made explicit in the prospective memory literature (but see [1], [21], [33]) and more often only briefly acknowledged, typically within the method section of the manuscript where it is easily missed. To illustrate, McDaniel et al.[7] explain “If a cue produces enough interaction with a memory trace, then the system delivers to awareness [consciousness] the information associated with the cue [previously formed plan]” (p. 606) and “the target event simply stimulates (or fails to stimulate) a reflexive-associative process that brings the intended action to awareness [consciousness] (p. 606). Marsh, Hicks, Hancock, and Munsayac [34] explain in the method section that “this task was merely a distractor task placed between the prospective instruction and the onset of the rating task so that the prospective task did not become vigilance task…” (p. 304). Similarly, Shapiro and Krisnan [35] note in the method section that “this delay [15 min] has been shown to be sufficient to clear short-term memory and to ensure that it is not treated as a vigilance task…” (p. 174). Thus, at present, only careful reading of the method section allows a reader to determine whether the report is about vigilance or about prospective memory proper.

In habitual prospective memory [1], [33], [36], as in prospective memory proper, a plan is made, leaves consciousness, and then must be brought back into consciousness at the right time and place, but in contrast to prospective memory proper, such a plan needs to be brought back to consciousness repeatedly at all times the prospective memory cue calls for the plan's performance.

### Prospective Memory Ability versus Task Performance

Prospective memory tasks are measurement tools that are used to make inferences about prospective memory abilities. The extent to which each individual's prospective memory task score reflects that individual's prospective memory ability, as opposed to measurement error or some other ability, depends critically on the reliability and validity of such measurement tools. Unfortunately, reliability and validity of prospective memory tasks as measures of prospective memory ability is rarely reported, considered, and discussed (but see [1], [12], [16], [37].

Two issues in the measurement of prospective memory ability suggest that evaluation of reliability and validity of various prospective memory measures is especially critical. First, prospective memory tasks typically utilize binary outcomes; that is, a participant either responds to a prospective memory cue (success) or does not (failure). When several minutes, hours, or days intervene between the prospective memory instructions and appearance of a prospective memory cue, task performance is likely to reflect prospective memory proper but this single binary outcome trial is inefficient and much less reliable than continuous indices used to measure retrospective memory [1], [12], [16]. In contrast, when many prospective memory cues are presented, for example, one cue every 30s for a total of 30 cues, the proportion of successes is more reliable than a single or a few cues (e.g., reliability improved from 0.12 with 6 cues to 0.62 with 30 cues in Kelemen et al. [37] using a task modeled after Einstein and McDaniel [4]) and the proportion can be treated as a continuous rather than discrete measure. However, the problem with using such a large number of cues is that the plan tends to remain in consciousness and the task then measures vigilance rather than prospective memory proper. Accordingly, the majority of indices of prospective memory proper used in previous research suffer from low reliability due to binary outcome measurement (but see [12], [16] for examples of highly reliable continuous indices of prospective memory proper).

Second, as illustrated by the example of buying groceries en route home, it is widely recognized that success on prospective memory tasks depends on two components: a prospective component (becoming aware of the plan at the right time and place) and a retrospective component (being able to recollect the content of the plan, e.g., what groceries to buy) [1], [4], [16], [33], [38]. Accordingly, when a prospective memory measure has a heavy retrospective memory component (e.g., when participants have to respond to 30 different prospective memory cues, that is, remember 30 cue-action pairs [39]), successful performance will depend more upon the retrospective rather than the prospective component, and the index will have low validity in measuring prospective memory ability [1], [16]. An even more extreme example is illustrated by Martin, Kliegel, and McDaniel's [40] study. According to the method section, when it was time to initiate the prospective memory plan, Martin et al. *told* participants that it was time to execute the prospective memory task (i.e., “participants not initiating the multitask prospective memory paradigm by themselves *were prompted by the experimenter* [emphasis added]”, p. 199). The participants' ability to recollect the previously formed plan (i.e., the number of prospective memory subtasks started) was then used as the index of prospective memory, even though this measure indexes primarily retrospective memory ability.

A number of researchers [1], [11], [38] have pointed out that the prospective memory component can be measured more directly by minimizing the retrospective memory component load and by requiring participants to respond with a simple action such as stopping in response to noticing the cue. This action of stopping is the best index of the prospective memory component and the least confounded by retrospective memory ability to recollect the content of the plan.

### Event-Cued versus Time-Cued Tasks

Harris [36] and other prospective memory researchers have made a distinction between event-cued and time-cued prospective memory tasks. In event-cued prospective memory tasks, a prospective memory cue is an event, such as passing a supermarket, whereas in time-cued prospective memory tasks, a prospective memory cue is time, such as 3 p.m.. However, a time cue can frequently be seen as an event cue or it can be translated into an event cue. To illustrate, a time cue is frequently accompanied by an event cue, for example, 9 p.m. is accompanied by sunset. In contrast, an event cue is often difficult, if not impossible, to translate to a time cue. Thus, we [1] have argued elsewhere that time may simply be a less intrusive cue than many event cues and the question whether time versus event-cued prospective memory is fundamentally different is not yet settled.

### Laboratory versus Naturalistic Tasks

It has been argued that people's behavior in laboratory conditions is not necessarily the same as in natural settings, and in turn, that research findings obtained with laboratory (artificial) tasks need not generalize to naturalistic tasks for a number of reasons, including lack of experimental control over naturalistic tasks and differential familiarity of participants with laboratory tasks. Indeed, early studies of prospective memory showed that older adults outperformed younger adults in natural settings [30] but that younger adults outperformed older adults in laboratory settings [38], the findings later supported by Birt's meta-analysis of prospective memory research findings [13] and confirmed by Henry et al. [14]. However, as noted above, this conclusion may be misleading if studies in laboratory versus naturalistic settings examined different aspects of prospective memory (e.g., event-cued versus time-cued prospective memory).

### Dichotomous versus Continuous Measurement of Prospective Memory Ability

In prospective memory and other research fields, continuous ability measures are very rare [1], [12] and dichotomous success/failure measures are prevalent, even though the underlying ability is continuous and true scores are most likely normally distributed. What is the effect of having only dichotomous or dichotomized measures on estimated standardized effect sizes used in previous meta-analyses of prospective memory? Dichotomization of continuous scores (true or observed ones) discards information about individual differences, measures individual differences with a greater degree of error, therefore, decreasing the reliability of measurement and, as discussed above, resulting in artificially lower effect sizes [41].

An even lesser known fact is that this decrease in reliability depends on the specific dichotomization point–the cutoff score where a continuous measure is dichotomized–and test difficulty when ability is measured using dichotomous success/failure outcome measures. Specifically, the observed effect size d_O_ = h/sqrt(p*q), where p is proportion of population above the cutoff point (proportion of successes), q is proportion of the population below the cut off point (proportion of failures), and h is ordinate of the normal curve at the point of dichotomization. Figure 4 and Table 2 illustrate the influence of dichotomization on effect size; dichotomization reduces the true effect size by at least 30% when p = q but by much more as the split becomes more uneven with reduction of 70% or more when the ratio of success to failures is 10:90 or more extreme.

**Figure 4:** Undesirable consequences of using *d* or *r*-to-*d* translational formulas with dichotomized performance indices. Panel A shows a hypothetical distribution of true ability scores in two groups–younger and older adults–when the true effect size is 1.0. Panel B shows the proportion of younger persons passing the test as a function of test difficulty–proportion of older persons passing the test–for three true effect sizes: 0.5 (dashed line closest to the diagonal), 1.0 (solid line), 1.5 (dashed line farthest from the diagonal), with diagonal representing the line of no age-differences in proportion of persons passing the test. Panel C show raw age decline as a function of older adults' performance; it demonstrates that as the test becomes easier and easier, the raw differences between proportions of younger and older persons diminish, clearly limited by the ceiling, the diagonal line indicating maximum possible age decline for a given level of older adults performance. Panel D shows observed d (calculated from phi) as a function of test difficulty (performance of older adults). Panel E show the underestimate of observed d as a proportion of true effect size d; for our example true effect size d = 1.0. Panel F shows the statistical power to detect true effect size d of 1.0 SD with 10, 30, and 100 participants, when using dichotomized measures, as a function of test difficulty. See Table 2 for numerical examples and the text for a more detailed explanation.

**Table 2:** Effect of dichotomization on various effect size indices when true effect size d = −1.0.

	Dichotomization point (z_young_)									
	2.5	−2	−1.5	−1.5	−0.5	0.0	0.5	1.0	1.5	2.0
p_young_	0.99	0.98	0.93	0.84	0.69	0.50	0.31	0.16	0.07	0.02
p_old_	0.93	0.84	0.69	0.50	0.31	0.16	0.07	0.02	0.01	0.00
n_young_ passed	99	98	93	84	69	50	31	16	7	2
n_old_ passed	93	84	69	50	31	16	7	2	1	0
n_young_ failed	1	2	7	16	31	50	69	84	93	98
n_old_ failed	7	16	31	50	69	84	93	98	99	100
p_old_-p_young_	−0.06	−0.14	−0.24	−0.34	−0.38	−0.34	−0.24	−0.14	−0.06	−0.02
d_phi_	−0.31	−0.50	−0.64	−0.77	−0.82	−0.77	−0.64	−0.50	−0.31	−0.20
d_p_	−0.31	−0.50	−0.64	−0.78	−0.82	−0.78	−0.64	−0.50	−0.31	−0.20
d_hh_	−1.11	−1.23	−0.98	−0.91	−0.88	−0.91	−0.98	−1.23	−1.11	-.–
d_probit_	−0.85	−1.06	−0.98	−0.99	−0.99	−0.99	−0.98	−1.06	−0.85	-.–

*Note.* This example assumes that n per group is 100.

Clearly, dichotomous measurement substantially underestimates the true population effect size and such underestimation is much more severe as the proportion of successes to failures is more extreme [41]. Thus, because effect size estimates underestimate true effect sizes much more for dichotomous than for continuous data, the effect of aging on prospective versus retrospective memory will appear smaller, and seemingly contradict Craik's [2], [3] theory, *solely due to differences in measurement methods* (dichotomous indices for prospective memory versus continuous indices for retrospective memory) rather than true differences in function.

### Effect Size Indices for Dichotomous Prospective Memory Data

Many handbooks on how to do meta-analysis focus on the most widely used index of effect size–the *standardized mean difference d* , the difference between means divided by the standard deviation. They offer various formulas on how to calculate *d* from means and *SD*s as well as from other statistics (i.e., *r*s, *t*s, *F*s, chi-squares) when means and *SD*s are not available. Similarly, many of these texts also discuss and provide various computational and translational formulas for an alternative effect size index *r* [42]. Moreover, these texts typically recommend the *phi* correlation coefficient as an effect size index that can be calculated over dichotomous outcome measures and easily translated to *d* using the same *d* from *r* formulas (e.g., [42]). However, others have pointed out that *d* and *r* are not necessarily the most appropriate indices of effect size, that selection of an effect size index has to consider limitations and assumptions of using each specific index, and that mindless use of *d* or *r* may lead to substantial inferential errors [43]. Specifically, the effect size *d*–difference between the means divided by the standard deviation–depends critically on several basic assumptions, most importantly that the means reflect true abilities and the standard deviations reflect true variability. To the extent to which these basic assumptions are violated, for example, because of ceiling and floor effects, the effect size *d* will lead to misleading results. Moreover, while *d* is an appropriate effect size metric for continuous measures, it severely underestimates the true effect size when it is used with dichotomized variables, that is, variables that are continuous in nature but are measured using dichotomous indices such as failure/success indices [43], [44].

Figure 4 and Table 2 demonstrate the undesirable consequences of using *d* or *r*-to-*d* translational formulas with dichotomized performance indices. Figure 4a shows the hypothetical distribution of true ability scores in two groups–younger and older adults. It shows that older adults perform 1 *SD* below younger adults, and thus, the size of this age decline in terms of *d* is 1.0. When this continuously distributed ability is measured using dichotomous success/failure measures, test difficulty determines the cut-off point. Sliding the cut-off point to the left makes the test easier whereas sliding the cut-off point to the right makes it more difficult. To illustrate, for a cut-off point set at *z* = −0.5 (relative to younger adults' mean), .69 of younger and .31 of older adults pass the test; for a cut-off point set at *z* = −.2, .98 of younger and .84 of older adults pass the test; and for a cut off point set at *z* = −3, .99 of younger and .98 of older adults pass the test (see Table 2). Figure 4b shows the proportion of younger persons passing the test as a function of the proportion of older persons passing the test for three true effect sizes: −0.5 (dashed line closest to the diagonal), −1.0 (solid line), −1.5 (dashed line farthest from the diagonal), with the diagonal representing the line of no age differences in proportion of persons passing the test. As the test becomes easier (or more difficult) the separation between the lines of different true effect sizes decreases. Figure 4c shows raw age declines as a function of older adults' performance; it demonstrates that as the test becomes easier, the raw differences between proportions of younger and older persons diminish, clearly limited by the ceiling, the diagonal line indicating maximum possible age decline for a given level of older adults' (lower scoring group's) performance.

Using *phi* and the usual *phi*-to-*d* transformation formula published in meta-analysis recipes [42], [45], the observed *d* based on the dichotomized data can be calculated as a function of test difficulty; panel D shows that the observed *d* severely underestimates the true effect size and that this underestimation is especially severe when the test is easy or very difficult. Figure 4e shows the underestimate of observed *d* as a proportion of true effect size *d*; for our example true effect size *d* = 1.0, the panel shows that observed *d* is underestimated by as much as 50% by the time performance of older adults reaches .80 and by as much as 60% by the time it reaches .90. This shows that researchers need to adjust test difficulty down to 0.2 to 0.4 (in terms of older adults' passing rate) to allow for their dichotomized success/failure indices to capture the largest portion of true effect size, and even then, the dichotomous measures will miss about 20% of true effect size, depending on the true effect size. In turn, Figure 4f shows the statistical power to detect the true effect size *d* of 1.0 *SD* with 10, 30, and 100 participants, when using dichotomized measures, as a function of test difficulty. A recent review of event-cued prospective memory demonstrated that many studies employed as few as 12 participants per age group and few employed more than 30 participants [16]. Clearly, studies that use only 12 participants per age group are so severely underpowered that, more often than not, one must find no age differences even though the true age effect size is large (i.e., 1.0 *SD*). Moreover, age differences are next to impossible to detect when the test is easy, when a substantial portion of lower scoring older adults pass the test and performance is limited by ceiling effects. Similarly, even studies with 30 participants remain severely underpowered when a dichotomous measure is too easy. To illustrate, when older adults performance is .80 and above, the power of the test is less than 50% to detect true age differences as large as *d* = 1.0. Finally, even with a massive true age decline of 1.5 *SD*, power drops well below the desirable .95 when performance of older adults surpasses 0.80.

What is then the best effect size index for dichotomous data? Theoretical analysis (see Figure 4) as well as recent Monte Carlo simulation evidence [43] suggest that *d* calculated from dichotomous data using observed means and *SD*s (denoted *d*_p_) as well as *d* from *phi* (*d_phi_*) are one of the worst effect size indices for dichotomous data as they underestimate the true effect size so severely. Several alternative indices are clearly preferable, including odds ratios (OR) and probit indices. Both of these indices allow easy translation to the effect size *d* equivalent (*d_hh_* for OR and *d_probit_* for probit) and underestimate the true effect size much less and only at much more extreme test difficulties than *d_p_ or d_phi_* [43]. The last four rows of Table 2 illustrate this point for our hypothetical example of true *d* = 1.0 and dichotomization points ranging from −2.5 to 2.0 relative to younger adults (with 100 participants in each age group). Whereas *d_p_ and d_phi_* range from a low of −.31 (for a dichotomization point set at z = −2.5) to a high of −0.82 (for z = −0.5) when true *d* is 1.0, *d_hh_* performs much better (ranging from −0.88 to −1.23) and *d_probit_* estimates the true effect size the best (ranging from −0.85 to −1.06).

An alternative and preferred solution is to use a model fitting approach to determine which effect size curve fits the data best. Specifically, the performance of younger adults can be plotted as a function of performance of older adults for all previous investigations (cf., L'Abbé plot [46]) and then find the best fitting theoretical effect size curve (see Figure 4b for examples) using double variate error minimization methods, either with or without weighting each point by its sample size. This modeling procedure will result in an unbiased estimate of true effect size, unaffected by ceiling effects, skewed standard deviations, low test reliability, and other distribution problems. Moreover, bootstrapping techniques can then be used to obtain 95% confidence intervals as well as test for differences between estimated *d*s between various subdomains [47]–[49].

### Shortcomings of Prospective Memory Research

Prospective memory researchers have been criticized for their failure to define and delineate that which they are studying [31], [32] (see also [1]). This criticism seems to be as true today as it was a decade ago. As pointed out above, the vast majority of definitions of prospective memory found in individual reports assume that widely discrepant tasks, such as monitoring a kettle and remembering to buy groceries en route home, measure the same unitary construct–the ability to remember to perform some planned action at the appropriate time in the future. However, mounting experimental evidence suggests that this assumption is unwarranted and that prospective memory, like retrospective memory, is comprised of several subdomains, and that the magnitude of age declines varies across the subdomains of prospective memory. If so, the controversy about the effects of aging on prospective memory may be entirely artificial, entirely due to researchers talking about different subdomains of prospective memory, one that shows small or minimal age differences and the other that shows large, substantial age declines. Moreover, averaging across the subdomains as if they did not exist is tantamount to taking watermelons, oranges, and grapes, averaging their weight, sizes, and flavors, and hoping that this will tell us something about fruit in general.

Equally importantly, any informative meta-analysis of prospective memory must take into account not only methodological problems afflicting large proportion of research in the area (ceiling effects, low reliability, age confounds) but also the dichotomous nature of the vast majority of prospective memory indices that render *d_p_* and *d_phi_* based indices inappropriate for the reasons discussed above.

### Transparent, Informative, and Robust Meta-Analysis of Prospective Memory and Aging

The present meta-analysis of previous prospective memory research has three aims. The first aim is to map out aspects of prospective memory that have been investigated versus aspects that have been largely ignored, by tabulating how many age contrasts fall in to each of the 12 cells formed by crossing prospective memory subdomain (prospective memory proper, vigilance, habitual prospective memory), cue type (event-cued versus time-cued), and experimental setting (laboratory versus naturalistic). The second aim is to determine if prospective memory declines with age, the pattern of any age declines across the adult lifespan (e.g., linear versus accelerated), and the extent to which the magnitude of age differences varies with prospective memory subdomain, cue type, experimental setting, as well as other design variables. Are some aspects of event-cued prospective memory spared by aging as claimed by some researchers? Are age declines in prospective memory proper larger than age declines in vigilance? Are age declines on laboratory tasks and age improvements on naturalistic tasks consistent across prospective memory subdomains (i.e., vigilance, prospective memory proper, habitual prospective memory)? The third aim is to compare the size of age declines in prospective memory to age declines in retrospective memory under controlled laboratory conditions. As noted above, Craik [2], [3] suggested that age declines on prospective memory are larger than on free recall. Given that age declines in recall are about 1 *SD* (*d* = 1.01 [23]; *d* = 0.97 [24]), if Craik is correct then we should observe age declines corresponding to *d* = 1.0 or more on prospective memory proper.

Importantly, to avoid biases and artificial reductions in estimated effect sizes arising from methodological and measurement issues with primary data including prevalent ceiling effects, low reliability, and dichotomous nature of prospective memory indices, the present article approaches this problem in three different ways: robust outcome count meta-analysis, graphical meta-analysis combined with effect size model fitting, and more traditional meta-analysis using d*_probit_* rather than the inferior d*_p_* and d*_phi_* based methods that derive *d* from means and *SD*s, or *t*s, *ps*, and *Fs*. The robust outcome count methods are simple, transparent, and persuasive, even if not as powerful as modeling or parametric approaches to meta-analysis. The graphical model fitting methods are powerful, transparent, and informative, and make obvious many fundamental problems with primary data including ceiling effects. The more traditional d*probit* meta-analysis will satisfy traditionalists even though traditional meta-analyses with *t*s, *p*s, and *Q*s are non-transparent, and if conducted without prior primary data checking, may easily lead to misleading conclusions and claims about prospective memory and aging.

## Materials and Methods

### Studies Included In Meta-Analysis

The search for relevant studies proceeded in several ways. First, the *PsycLIT* database was searched, from the earliest available date to the end of June 2007, for the following terms: “prospective memory” and “memory for intentions”. Second, the references in all relevant articles and book chapters, retrieved by any method, were examined for potentially relevant articles and the identified articles were examined for relevance. Third, the references in Henry et al. [14] and Birt [13] were examined for potentially relevant articles and these were examined for relevance.

#### Inclusion and Exclusion Criteria

*A*ll studies that reported performance on prospective memory task for at least one group of younger and one group of older adults; were healthy and without any diseases known to affect cognition (e.g., dementia); provided at least mean performance for each age group; and were written in English were included in the review. For several studies with more than two age groups spanning adult lifespan (e.g.,[38], [50]–[52]), the groups younger than 60 years of age were collapsed into younger group and the groups older 60 years of age were collapsed into older group.

Tasks were considered to be prospective memory tasks if they required participants to perform some action in the future without any prompting from experimenters. This definition excluded the ostensibly prospective memory studies by Martin et al. [40] and Kliegel, Martin,and Moor [53] as participants in these studies were reminded when it was time to start performing the prospective memory plan, and thus, the “prospective memory” score reflected only retrospective memory–the total number of actions remembered.

#### Final Sample of Studies

The final sample included 60 reports consisting of 233 experimental conditions comparing younger and older adults' performance.

### Recorded Variables

For each age contrast, the recorded variables included authors; year of publication; prospective memory subdomain (prospective memory proper, vigilance, habitual prospective memory); prospective memory cue type (event versus time); experimental setting (lab versus natural); type of ongoing task; experimental condition; number of participants in each age group; mean performance and standard deviation for each age group (if available); duration of prospective memory instructions to prospective memory task delay; prospective memory performance scoring method (lenient or strict); the number of prospective memory cue-action associations that participants were required to remember; the number of different cues presented to each participant; the number of prospective memory cues (same and different) presented to each participant; the modality of prospective memory cue (visual, auditory); and reliability of prospective memory measures (if reported).

#### Laboratory versus Naturalistic prospective memory Tasks

Experimenter designed controlled laboratory tasks were classified as laboratory tasks whereas tasks performed during the course of participants' normal daily activities (e.g., sending a postcard, calling back at a pre-arranged time) were classified as naturalistic tasks.

#### Event-cued Prospective Memory v. Time-cued Prospective Memory

Consistent with the definitions outlined above, each prospective memory task was classified as measuring event-cued prospective memory (EC ProM) if a task required a response to an event cue and as measuring time-cued prospective memory (TC ProM) if the task required a response at a specific time. As noted above, however, some nominally TC prospective memory tasks may be converted by participants to EC ProM tasks if task conditions allow such conversion [1].

#### Prospective Memory Proper, Vigilance, and Habitual Prospective Memory

Following the definitions above, each prospective memory task was classified as measuring prospective memory proper (ProMP), vigilance, or habitual prospective memory (HProM). Tasks that included a time delay or intervening task between prospective memory instructions and commencement of an ongoing task (I-T delay) were classified as measuring prospective memory proper whereas tasks that included no I-T delay were classified as measuring vigilance. If a prospective memory proper task was to be executed repeatedly (with the plan likely to leave consciousness between successive presentations of prospective memory cues), it was classified as a habitual prospective memory task (HProM). While Einstein, McDaniel, Smith, and Shaw [54] claimed that they measured habitual prospective memory, the cue-to-cue delay between presentations of successive cues in this “habitual” prospective memory task was only 3–4 minutes, and therefore, the plan likely remained in consciousness and the task did not index habitual prospective memory, and moreover, because Einstein et al. did not include any delay between prospective memory instructions and the start of the ongoing task, their study most likely measured vigilance. Consistent with this analysis, Einstein, McDaniel, Richardson, Guynn, and Cunfer [55] themselves believed that they measured vigilance or prospective memory proper rather than habitual prospective memory even though they used multiple cues and much longer cue-to-cue delays of 7 minutes in one of their prior studies.

#### Age-Related Design Confounds

A careful review of methods as well as published critiques of prospective memory research reveals that a large number conditions included age-related design confounds. Accordingly, each condition was categorized into one of the four age-confound categories: no age-confound, confound favoring old, confound favoring young, and confounds with unknown effect. Confounds favoring old are primarily of the two kinds: *ongoing task confounds* and *participants' intelligence confounds*.

*Ongoing task confounds favoring older adults* were originally introduced by Einstein and McDaniel [4] who made the ongoing task easier for older than for younger adults and these confounded designs were later adopted by a number of investigators who followed in their steps. Because a number of studies have shown that higher ongoing task demands reduce prospective memory performance, making the ongoing task easier for older adults artificially reduces the size of age differences in prospective memory performance and makes it impossible to disentangle effects of aging from effects of giving older adults easier ongoing task.

*Participant intelligence confounds favoring older adults* are found in the studies by Einstein and McDaniel [4], Cherry and LeCompte [56], Reese and Cherry [57], Cheery and Plauche [58], [59] who compared very intelligent older adults with less intelligent younger adults. Since intelligence is positively correlated with prospective memory performance [12], [56], [60], as well as with many other cognitive tasks, this confound artificially reduces the size of age differences in prospective memory performance. To illustrate, Cherry and LeCompte [56] claimed that age differences were absent when high ability young and older adults were compared. However, this is not at all surprising since “high ability” older adults scored almost 2 *SD* higher than “high ability” younger adults on a verbal intelligence test. For purposes of this article, the data are considered confounded with intelligence if older adults score more than 1 *SD* above the ability of younger adults (e.g., [4], [56]–[58]).

*Confounds favoring younger adults* involve designs that included older participants who were afflicted by various diseases known to negatively affect cognition. To illustrate, Mantyla and Nilsson [61] conducted a population-based study of prospective memory and inspection of participants characteristics reveals that many participants scored within the impaired range on the Mini Mental State Examination (Folstein, Folstein, & McHugh, 1975) that serves as a quick index of possible dementia.

*Confounds with unknown effects* include conditions where participants' prospective memory task was to ask for their belongings at the end of the experiment and different participants gave experimenters different items [40], [62], [63].

#### Low versus High Retrospective Memory Load

It is widely acknowledged that performance on prospective memory tasks is a composite of prospective memory and retrospective memory abilities [1], [38], [64]. To illustrate, McDermott & Knight [39] required participants to remember and to respond to 30 different cues with 30 different actions. However, normal healthy adults are typically unable to remember 30 cue-action pairs [15]. Thus, when a task depends heavily on retrospective memory abilities, performance on the task may depend more on well-documented age declines in retrospective memory than on age declines in prospective memory. In contrast, when participants are required to respond to only one cue with one specific action, performance on the task will depend primarily on prospective memory ability rather than retrospective memory ability. For this reason, the coded variables included the number of unique prospective memory cue-action pairs that were part of the prospective memory plan.

#### Lenient versus strict scoring

Dobbs and Rule [38] were the first to attempt to disentangle the prospective from the retrospective component and they proposed that participants' awareness that something had to be done in response to the prospective memory cue was a more pure index of prospective memory than participants' correct performance of the previous plan, as such an index places minimal requirements on participants' retrospective memory abilities. Accordingly, prospective memory scores were classified as lenient if participants merely needed to remember that something was to be done and strict if they needed to accurately execute the plan to be successful on the prospective memory task [1].

#### Focal versus Non-Focal Cues

Einstein and McDaniel made a distinction between focal versus non-focal prospective memory cues and proposed that performance on prospective memory tasks with focal cues is unaffected by aging because retrieval of the previous plan is “reflexive” upon appearance of such focal cues[6]. They defined focal cues are cues that participants must work with whereas non-focal cues are cues that need not be processed by participants during the course of the ongoing task. By this definition, a questionnaire a participant is required to fill in is considered a focal cue if prospective memory instructions require the participant to perform some planned action when they are presented with the questionnaire and required to fill it in. Accordingly, we should see no age declines on this relatively frequently used prospective memory proper task (e.g., [11], [12], [38], [50], [51]). In contrast, the color of a toy is considered a non-focal cue when the ongoing task requires participants to sort toys into several semantic categories and does not require them to attend to each toy's color. Thus, for each task, prospective memory cues were classified as focal or non-focal.

#### Multiple Effect Sizes from Single Studies

Effect sizes were calculated for each age contrast, that is, for each reported condition with both young and older adults. However, to satisfy an independence assumption for application of meta-analysis, each participant could contribute to only one age contrast for statistical analysis purposes. Thus, when one group of participants was tested under 4 different conditions, the following criteria were used to select the condition used in the statistical analyses: (1) condition which was administered first was preferred (e.g., name task was used from Uttl et al. [11]; block 1 was chosen from Maylor [65]); (2) condition with smaller retrospective memory load was preferred; (3) condition with lenient scoring was preferred; and (4) if the preceding criteria were insufficient to unambiguously chose a condition, the condition was selected randomly.

#### Data Visualization and Modeling, Robust Techniques, and Conventional Meta-Analysis

To avoid unwarranted conclusions and to ensure high confidence in the findings, the primary data were analyzed in three ways. First, data visualization and modeling techniques were employed to determine unbiased effect size estimates unaffected by ceiling effects, skewed standard deviations, and other distribution problems that are widespread in prospective memory research [15], [16]. To this end, for each prospective memory subdomain (prospective memory proper, vigilance, habitual prospective memory), prospective memory cue type (event-cued versus time-cued), and study setting (lab versus naturalistic), performance of younger adults was plotted as a function of performance of older adults and then the best fitting theoretical effect size curve and associated effect size were determined using double variate squared error minimization methods, both with and without weighting each point by its sample size. An added advantage of this methodology is that it minimizes the influence of ceiling-limited data as data points close to either the floor or ceiling have minimal or no effect on the determination of the best fitting curve. The 95% CI on fitted effect sizes were derived and the differences between the effect sizes were tested using bootstrapping methods that are robust, conservative, and require fewer assumptions than classical methods[47].

Second, for each prospective memory subdomain, prospective memory cue type, and study setting, robust statistical techniques–counts and sign tests–were used to determine if the specific prospective memory subdomain is or is not affected by aging.

Third, for each prospective memory subdomain, prospective memory cue type, and study setting, conventional meta-analytic techniques were used to estimate effect sizes. However, given the dichotomous nature of primary outcome measures in all but a few studies (e.g., [12]), the probit was chosen as an effect size index and then transformed to *d*-equivalent *d_probit_*. Both theoretical and empirical simulation research as well as the examples in Table 2 show that *d_probit_* underestimates the true effect size much less than *phi* to *d* transformations or *d_p_* indices used in previous meta-analyses of prospective memory when primary performance indices are dichotomous. Even though these results are not reported, the data were also analyzed using odds ratios and the odds ratio analyses yielded nearly identical effect sizes.

To take into account the methodological quality of primary data and to avoid misleading and biased results, the studies with age-related confounds were blocked by confound type (intelligence, ongoing task difficulty) and analyzed separately.

## Results

The search identified 60 articles with 233 age contrasts (see Tables 3–[Table pone-0001568-t004] [Table pone-0001568-t005] [Table pone-0001568-t006] 7), representing 10,578 younger (mean age = 25.1 years, *SD* = 11.00) and 6,379 older (mean age = 71.3 years, *SD* = 5.07) individuals*conditions, almost tripling the size of the meta-analysis reported by Henry et al. (2004). Henry et al. (2004) identified only 26 articles with 83 age contrasts, primarily because they did not conduct a comprehensive search for all relevant studies (e.g., they excluded studies published in book chapters, e.g., [11], [30]) and because a number of articles were published after the cut-off date for their meta-analysis (December 2001). Thus, in term of accumulated research, the articles reviewed in the present meta-analysis represent substantial advance over previous meta-analyses (e.g., Birt [13]; Henry et al. [14]) and represent over 25 years of research on prospective memory and aging.

**Table 3:** Confound-free Prospective Memory Proper Age Contrasts in Laboratory Settings by Cue Type (Event, Time).

First Author & Year	Exp. no.	Condition	Ongoing Task	No. cues	# Cue-Action pairs	Lenient/Strict Scoring	Young n	Older n	ProM Young M	ProM Older M	ProM Age Effect	Confounds
**EC ProMP**												
*Continuous indices of ProMP (higher mean represents poorer ProMP)*												
Graf '02*[70]	1	visual	A/B Card Sorting	1	1	L	60	51	8.53	10.19	-	
Uttl '06*[12]	1	visual	A/B Card Sorting	1	1	L	29	18	9.97	15.53	-	
Uttl '06*[12]	1	auditory	A/B Card Sorting	1	1	L	29	18	7.06	15.05	-	
*Dichotomous indices of ProMP (proportion correct)*												
Cuttler '07 [51]	1	questionnaire	u/t	1	1	S	110	31	0.85	0.73	-	
Cuttler '07 [51]	1	plug in phone	u/t	1	1	S	110	31	0.49	0.22	-	
Dobbs '87 [38]	1	ask for pen	u/t	1	1	S	138	61	0.97	0.84	-	
Ducheck '06 [80]	1	knowledge	knowledge	8	1	S	20	33	0.87	0.69	-	
Kliegel '00[63]	1	six elements	u/t	1	1	S	31	31	0.64	0.36	-	
Kliegel '04 [81]	1	six elements	u/t	1	1	S	19	21	0.95	0.33	-	
Salthouse '04[50]	1	red pencil	u/t	6	1	S	255	75	0.83	0.43	-	
Rendell '99 [82]	3	note-finish	u/t	1	1	L	175	80	0.78	0.21	-	
Tombaugh '95 [29]	1	6 tasks	u/t	6	6	S	31	33	0.87	0.60	-	
Uttl '01 [11]	1	name	u/t	1	1	L	31	23	0.84	0.43	-	
Uttl '01 [11]	1	letter	u/t	1	1	L	31	23	0.94	0.70	-	
Uttl '01 [11]	1	check	u/t	1	1	L	31	23	0.97	0.78	-	
West '88 [83]	2	message	u/t	1	1	S	26	26	0.85	0.50	-	
West '88 [83]	2	check & ask	u/t	1	1	S	26	26	0.81	0.31	-	
Zimmerman'05 [68]	1	identity	identity	4	1	S	80	40	0.98	0.78	-	
**TC ProMP**												
Rendell '99 [82]	3	stop-clock	u/t	1	1	S	175	80	0.65	0.20	-	

*Note.* Confounds: o  =  ongoing task was easier for older adults; i  =  older adults were substantially more intelligent than younger adults; dem  =  older group had higher proportion of participants who scored in dementia range on screening tests; e(6y, 23o)  =  exclusion of subjects (6 young, 23 old) for various reasons; ep (0y,5o)  =  exclusion of subjects (0 young, 5 old) because of low ProM performance; item  =  participants were to request a personal item back but the items varied from participant to participant; #cues  =  number of ProM cues varied from participant to participant.

Ongoing task: u/t  =  unrelated tasks; Q&A  =  questions and answers; PA  =  paired associates; WM  =  working memory; E&M STM  =  Einstein & McDaniel Short Term Memory task (WM task); WML3  =  working memory task; WMLVar  =  working memory task.

a Patton'93: ProM task was “to shut off the movie after exactly 30 min had elapsed”. However, the article reports only deviation from target shut off time in s. Since the article does not mention that any participants forget to shut off the movie, it is assumed that all did.

**Table 4 pone-0001568-t004:** Confound-free Vigilance Age Contrasts in Laboratory Settings by Cue Type (Event, Time).

First Author & Year	Exp. no.	Condition	Ongoing Task	No. cues	# Cue-Action pairs	Lenient/Strict Scoring	Young n	Older n	ProM Young M	ProM Older M	ProM Age Effect	Confounds
**EC Vigilance**												
Cohen '01 [84]	1	very related	PA	24	24	L	24	24	0.92	0.78	-	
Cohen '01 [84]	1	somewhat related	PA	24	24	L	24	24	0.87	0.72	-	
Cohen '01 [84]	1	unrelated	PA	24	24	L	24	24	0.73	0.52	-	
Cohen '01 [84]	2	picture+word related	PA	24	24	L	24	24	0.96	0.85	-	
Cohen '01 [84]	2	picture+word unrelated	PA	24	24	L	24	24	0.91	0.74	-	
Cohen '01 [84]	2	word only related	PA	24	24	L	24	24	0.74	0.45	-	
Cohen '01 [84]	2	word only unrelated	PA	24	24	L	24	24	0.73	0.34	-	
Cohen '03 [85]	1	none displaced	visual search	12	2	L	30	30	0.82	0.53	-	
Cohen '03 [85]	1	target displaced	visual search	12	2	L	30	30	0.71	0.54	-	
Cohen '03 [85]	1	cue displaced	visual search	12	2	L	30	30	0.80	0.59	-	
Cohen '03 [85]	2	cue displaced	visual search	12	2	L	31	32	0.56	0.45	-	
Cohen '03 [85]	2	target displaced	visual search	12	2	L	31	32	0.61	0.52	-	
Cohen '03 [85]	2	cue displaced	visual search	12	2	L	31	32	0.71	0.69	-	
Cohen '03 [85]	2	cue displaced	visual search	12	2	L	31	34	0.56	0.45	-	
Cohen '03 [85]	2	target displaced	visual search	12	2	L	31	34	0.61	0.39	-	
Cohen '03 [85]	2	cue displaced	visual search	12	2	L	31	34	0.71	0.55	-	
Einstein '95 [55]	2	specific cue	WM	3	3	S	11	12	0.85	0.83	-	
Einstein '95 [55]	2	general cue	WM	3	3	S	11	12	0.56	0.47	-	
Costermans ‘99 [86]	1	cp	movie	6	1	S	10	10	0.78	0.69	-	
Costermans ’99 [86]	1	vp/d = 7	movie	4	1	S	10	10	0.80	0.80	=	
Costermans ’99 [86]	1	vp/d = 3	movie	4	1	S	10	10	0.75	0.67	-	
Einstein '95 [55]	2	general cue	WM	3	3	S	12	12	0.56	0.47	-	
Einstein '97 [20]	1	standard	w/rating	6	1	S	16	16	0.71	0.53	-	
Einstein '97 [20]	1	demanding	w/rating+digit detect.	6	1	S	16	16	0.58	0.25	-	
Einstein '97 [20]	2	enc std/ret std	w/rating	6	1	S	16	16	0.66	0.58	-	
Einstein '97 [20]	2	enc std/ret dem	w/rating+digit detect.	6	1	S	16	16	0.64	0.38	-	
Einstein '97 [20]	2	enc dem/ret std	w/rating	6	1	S	16	16	0.47	0.54	+	
Einstein '97 [20]	2	enc dem/ret dem	w/rating+digit detect.	6	1	S	16	16	0.55	0.17	-	
Einstein '98 [54]	1	std att/no cue	u/t	11	1	S	15	15	0.91	0.69	-	
Einstein '98 [54]	1	std att/cue	u/t	11	1	S	15	15	0.89	0.73	-	
Einstein '98 [54]	1	div att/no cue	u/t	11	1	S	15	15	0.82	0.62	-	
Einstein '98 [54]	1	div att/cue	u/t	11	1	S	15	15	0.81	0.52	-	
d'Ydewalle '99 [87]	1	q&a	q&a	3	1	S	30	30	0.81	0.42	-	
d'Ydewalle '99 [87]	1	faces	face identification	3	1	S	30	30	0.92	0.73	-	
d'Ydewalle '01 [88]	1	low complexity	math	5	1	S	12	12	0.62	0.17	-	
d'Ydewalle '01 [88]	1	high complexity	math	5	1	S	12	12	0.70	0.73	+	
Kidder '97 [18]	1	WM 2/ProM 1	WM	6	1	S	15	15	0.98	0.98	=	e(6y,23o)
Kidder '97 [18]	1	WM 3/ProM 1	WM	6	1	S	15	15	0.82	0.69	-	e(6y,23o)
Kidder '97 [18]	1	WM 2/ProM 3	WM	6	3	S	15	15	0.97	0.85	-	e(6y,23o)
Kidder '97 [18]	1	WM 3/ProM 3	WM	6	3	S	15	15	0.90	0.63	-	e(6y,23o)
Logie '04 [89]	1	low arithmetic	movie+arithmetics	5	1	S	10	10	1.00	0.98	-	
Logie '04 [89]	1	high arithmetic	movie+arithmetics	5	1	S	10	10	0.96	0.80	-	
Mantyla '93 [90]	1	typical/primed	generate associates	8	4	S	16	16	0.86	0.75	-	
Mantyla '93 [90]	1	typical/nonprime	generate associates	8	4	S	16	16	0.80	0.49	-	
Mantyla '93 [90]	1	atypical/primed	generate associates	8	4	S	16	16	0.80	0.30	-	
Mantyla '93 [90]	1	atypical/nonprime	generate associates	8	4	S	16	16	0.48	0.22	-	
Mantyla '94 [91]	1	typical	generate associates	8	4	S	18	18	0.79	0.65	-	
Mantyla '94 [91]	1	atypical	generate associates	8	4	S	18	18	0.65	0.26	-	
Martin '03 [40]	1	word rating	w/rating	4	1	S	40	40	0.95	0.79	-	
Maylor '93 [92]	1	block 1	face identification	8	2	L	43	43	0.69	0.68	-	
Maylor '93 [92]	1	block 2	face identification	8	2	L	43	43	0.83	0.66	-	
Maylor '93 [92]	1	block 3	face identification	8	2	L	43	43	0.87	0.69	-	
Maylor '93 [92]	1	block 4	face identification	8	2	L	43	43	0.92	0.71	-	
Maylor '96 [60]	1	block 1	face identification	8	1	S	56	59	0.57	0.26	-	
Maylor '96 [60]	1	block 2	face identification	8	1	S	56	59	0.65	0.25	-	
Maylor '96 [60]	1	block 3	face identification	8	1	S	56	59	0.67	0.27	-	
Maylor '96 [60]	1	block 4	face identification	8	1	S	56	59	0.60	0.28	-	
Maylor '98 [65]	1	block 1	face identification	8	1	S	45	59	0.65	0.26	-	
Maylor '98 [65]	1	block 2	face identification	8	1	S	45	59	0.75	0.25	-	
Maylor '98 [65]	1	block 3	face identification	8	1	S	45	59	0.81	0.26	-	
Maylor '98 [65]	1	block 4	face identification	8	1	S	45	59	0.84	0.28	-	
Maylor '02 [93]	1	movie	movie	5	1	S	15	15	1.00	0.92	-	
Maylor '02 [93]	2	related	movie	5	1	S	10	10	1.00	0.88	-	
Maylor '02 [93]	2	unrelated	movie	5	1	S	10	10	0.96	0.90	-	
McDermott '04 [39]	1	movie	25-min video	27	27	L	30	30	0.73	0.58	-	
Park '97 [19]	1	6-event	WML3	6	1	S	16	16	0.94	0.71	-	
Park '97 [19]	1	12-event	WML3	12	1	S	16	16	0.92	0.87	-	
Rendell '00 [94]	1	irregular tasks	virtual week	70	6	L	20	20	0.78	0.42	-	
Rendell '00 [94]	1	regular tasks	virtual week	70	6	L	20	20	0.93	0.82	-	
Salthouse '04 [50]	1	concepts	concept ident.	4	1	S	255	75	0.75	0.49	-	
Salthouse '04 [50]	1	pictures	pictures task	9	1	S	255	75	0.95	0.81	-	
Salthouse '04 [50]	1	WML3	WML3	24	1	S	255	75	0.84	0.60	-	
Vogels '02 [95]	1	block 1	letter-monitoring	12	2	S	16	16	0.81	0.81	=	
Vogels '02 [95]	1	block 2	letter-monitoring	12	2	S	16	16	0.91	0.88	-	
Vogels '02 [95]	1	block 3	letter-monitoring	12	2	S	16	16	0.94	0.97	+	
Vogels '02 [95]	1	word comp	word-comparison	20	2	S	16	11	0.94	0.68	-	ep(0y,5o)
Vogels '02 [95]	1	pictures	pictures task	35	1	S	16	14	0.84	0.69	-	ep(0y,2o)
Vogels '02 [95]	1	no feedback	three-in a row task	36	1	S	15	13	0.84	0.86	+	ep(1y,3o)
Vogels '02 [95]	1	feedback	three-in a row task	36	1	S	15	13	0.88	0.87	-	ep(1y,3o)
West '99a [96]	1	w/classification	w/class category	20	2	S	24	24	0.96	0.79	-	
West '99a [96]	2	w/classification	w/class category	10	2	S	12	12	0.91	0.75	-	
West '03 [97]	1	w/classification	w/class	48	1	S	16	16	0.73	0.46	-	
West '01 [98]	1	w/classification	w/class.	40	1	S	16	16	0.95	0.83	-	
West '01 [10]	1	percep/immed	w/class color	16	4	S	20	20	0.86	0.60	-	
West '01 [10]	1	sem/immed	w/class color	16	4	S	20	20	0.41	0.24	-	
West '01 [10]	1	percept/post	w/class color	16	4	S	20	20	0.58	0.24	-	
West '01 [10]	1	sem/post	w/class color	16	4	S	20	20	0.28	0.19	-	
West '01 [10]	1	percep/immed	w/class category	16	4	S	20	20	0.89	0.58	-	
West '01 [10]	1	sem/immed	w/class category	16	4	S	20	20	0.58	0.39	-	
West '01 [10]	1	percept/post	w/class category	16	4	S	20	20	0.78	0.38	-	
West '01 [10]	1	sem/post	w/class category	16	4	S	20	20	0.64	0.24	-	
West '01 [10]	2	percep	w/class color	16	2	S	12	12	0.88	0.67	-	
West '01 [10]	2	seman	w/class color	16	2	S	12	12	0.70	0.41	-	
West '01 [10]	2	percept	w/class category	16	2	S	12	12	0.92	0.70	-	
West '01 [10]	2	seman	w/class category	16	2	S	12	12	0.92	0.73	-	
**TC Vigilance**												
d'Ydewalle '95 [99]	1	involving	movie	14	1	S	12	18	1.00	1.00	=	e(4y,4o)
d'Ydewalle '95 [99]	1	boring	movie	14	1	S	11	17	1.00	1.00	=	e(4y,4o)
d'Ydewalle '99 [87]	1	q&a	q&a	3	3	S	30	30	0.87	0.68	-	
d'Ydewalle '99 [87]	1	faces	face identification	3	3	S	30	29	0.97	0.88	-	
d'Ydewalle '01 [88]	1	low complexity	math	5	5	S	12	12	0.64	0.40	-	
d'Ydewalle '01 [87]	1	high complexity	math	5	5	S	12	12	0.61	0.10	-	
Einstein '95 [55]	1	WM	WM	2	1	S	12	12	0.92	0.63	-	
Logie '04 [89]	1	low arithmetic	movie+arithmetics	5	1	S	10	10	1.00	1.00	=	
Logie '04 [89]	1	high arithmetic	movie+arithmetics	5	1	S	10	10	0.96	0.84	-	
Martin '01 [100]	1	low complexity	Mastermind	6	1	S	30	30	0.92	0.67	-	
Martin '01 [100]	1	medium complexity	Mastermind	6	1	S	30	30	0.75	0.50	-	
Martin '01 [100]	1	high complexity	Mastermind	6	1	S	30	15	0.65	0.02	-	
Martin '03 [40]	1	w/rating	w/rating	4	1	S	40	40	0.97	0.74	-	
Maylor '02 [93]	1	movie	movie	5	1	S	15	15	1.00	0.70	-	
McDermott '04 [39]	1	movie	25-min video	1	1	S	30	30	0.97	0.67	-	
Park '97 [19]	2	6- or 12-intervals	WML3	9	1	S	32	32	0.63	0.34	-	
Park '97 [19]	2	6- or 12-intervals	none	9	1	S	24	24	0.80	0.58	-	
Patton '93 [101] a	1	stop video	movie	1	1	S	24	17	1.00	1.00	=	
Rendell '00 [94]	1	time check	virtual week	70	6	L	20	20	0.72	0.34	-	

*Note.* Confounds: o  =  ongoing task was easier for older adults; i  =  older adults were substantially more intelligent than younger adults; dem  =  older group had higher proportion of participants who scored in dementia range on screening tests; e(6y, 23o)  =  exclusion of subjects (6 young, 23 old) for various reasons; ep (0y,5o)  =  exclusion of subjects (0 young, 5 old) because of low ProM performance; item  =  participants were to request a personal item back but the items varied from participant to participant; #cues  =  number of ProM cues varied from participant to participant.

Ongoing task: u/t  =  unrelated tasks; Q&A  =  questions and answers; PA  =  paired associates; WM  =  working memory; E&M STM  =  Einstein & McDaniel Short Term Memory task (WM task); WML3  =  working memory task; WMLVar  =  working memory task.

a Patton'93: ProM task was “to shut off the movie after exactly 30 min had elapsed”. However, the article reports only deviation from target shut off time in s. Since the article does not mention that any participants forget to shut off the movie, it is assumed that all did.

**Table 5 pone-0001568-t005:** Confound-free Prospective Memory Proper Age Contrasts in Natural Settings by Cue Type (Event, Time).

First Author & Year	Exp. no.	Condition	Ongoing Task	No. cues	# Cue-Action pairs	Lenient/Strict Scoring	Young n	Older n	ProM Young M	ProM Older M	ProM Age Effect	Confounds
**EC ProMP**												
Dobbs '87 [38]	1	date questionnaire	u/t	1	1	L	138	61	0.50	0.25	-	
Rendell '00 [94]	2	irregular/event	actual week	70	10	S	16	16	0.66	0.83	+	
**TC ProMP**												
Cuttler '07 [51]	1	conference call	u/t	1	1	S	110	31	0.55	0.73	+	
Devolder '90 [102]	1	prediction	u/t	8	1	S	24	24	0.56	0.86	+	
Devolder '90 [102]	1	postdiction	u/t	8	1	S	24	24	0.57	0.81	+	
Kvavilashvili'07 [103]	1	call in	u/t	1	1	S	36	38	0.68	0.81	+	
Levy '80 [69]	1	appointment	u/t	1	1	S	86	45	0.55	0.67	+	
Martin '86 [104]	2	appointment	u/t	1	1	S	30	30	0.96	0.99	+	#cues
Rendell '99 [82]	1	diff./reg.	u/t	28	28	S	30	20	0.36	0.72	+	
Rendell '99 [82]	1	diff./irreg.	u/t	28	28	S	30	20	0.41	0.68	+	
Rendell '00 [94]	2	irregular/time	actual week	70	10	S	16	16	0.36	0.55	+	
Rendell '00 [94]	2	time check	actual week	70	10	S	16	16	0.24	0.26	+	
West '88 [83]	1	message	u/t	1	1	S	24	24	0.79	0.88	+	
West '88 [83]	1	mail postcard	u/t	1	1	L	24	24	0.92	0.96	+	

*Note.* Confounds: o  =  ongoing task was easier for older adults; i  =  older adults were substantially more intelligent than younger adults; dem  =  older group had higher proportion of participants who scored in dementia range on screening tests; e(6y, 23o)  =  exclusion of subjects (6 young, 23 old) for various reasons; ep (0y,5o)  =  exclusion of subjects (0 young, 5 old) because of low ProM performance; item  =  participants were to request a personal item back but the items varied from participant to participant; #cues  =  number of ProM cues varied from participant to participant.

Ongoing task: u/t  =  unrelated tasks; Q&A  =  questions and answers; PA  =  paired associates; WM  =  working memory; E&M STM  =  Einstein & McDaniel Short Term Memory task (WM task); WML3  =  working memory task; WMLVar  =  working memory task.

a Patton'93: ProM task was “to shut off the movie after exactly 30 min had elapsed”. However, the article reports only deviation from target shut off time in s. Since the article does not mention that any participants forget to shut off the movie, it is assumed that all did.

**Table 6 pone-0001568-t006:** Confound-free Habitual Prospective Memory Age Contrasts in Natural Settings by Cue Type (Event, Time).

First Author & Year	Exp. no.	Condition	Ongoing Task	No. cues	# Cue-Action pairs	Lenient/Strict Scoring	Young n	Older n	ProM Young M	ProM Older M	ProM Age Effect	Confounds
**EC Habitual**												
Rendell '00 [94]	2	regular/event	actual week	70	10	S	16	16	0.85	0.95	+	
**TC Habitual**												
d'Ydewalle '96 [105]	1	internal reminders	u/t	5	1	S	11	7	0.80	0.92	+	
d'Ydewalle '96 [105]	1	external reminders	u/t	5	1	S	3	6	0.96	0.98	+	
d'Ydewalle '96 [105]	2	internal reminders	u/t	5	1	S	15	15	0.84	0.94	+	
d'Ydewalle '96 [105]	2	external reminders	u/t	5	1	S	15	15	0.79	0.92	+	
d'Ydewalle '96 [105]	2	free to choose	u/t	5	1	S	15	15	0.69	0.84	+	
Moscovitch '82 [30]	1	call in	u/t	14	1	S	10	10	0.20	0.90	+	
Patton '93 [101]	1	mail postcards	u/t	4	1	S	24	17	0.72	1.00	+	
Patton '93 [101]	3	mail postcards	u/t	4	1	S	22	20	0.79	1.00	+	
Rendell '93 [28]	1	four times a day	u/t	56	4	S	32	58	0.49	0.70	+	
Rendell '93 [28]	1	once a day	u/t	7	1	S	32	58	0.47	0.72	+	
Rendell '99 [82]	1	same/reg.	u/t	28	4	S	30	20	0.32	0.71	+	
Rendell '99 [82]	1	same/irreg.	u/t	28	4	S	30	20	0.40	0.68	+	
Rendell '99 [82]	2	alarm	u/t	28	4	S	30	20	0.60	0.86	+	
Rendell '99 [82]	2	choice	u/t	28	4	S	30	20	0.42	0.78	+	
Rendell '00 [94]	2	regular/time	actual week	70	10	S	16	16	0.51	0.74	+	

*Note.* Confounds: o  =  ongoing task was easier for older adults; i  =  older adults were substantially more intelligent than younger adults; dem  =  older group had higher proportion of participants who scored in dementia range on screening tests; e(6y, 23o)  =  exclusion of subjects (6 young, 23 old) for various reasons; ep (0y,5o)  =  exclusion of subjects (0 young, 5 old) because of low ProM performance; item  =  participants were to request a personal item back but the items varied from participant to participant; #cues  =  number of ProM cues varied from participant to participant.

Ongoing task: u/t  =  unrelated tasks; Q&A  =  questions and answers; PA  =  paired associates; WM  =  working memory; E&M STM  =  Einstein & McDaniel Short Term Memory task (WM task); WML3  =  working memory task; WMLVar  =  working memory task.

a Patton'93: ProM task was “to shut off the movie after exactly 30 min had elapsed”. However, the article reports only deviation from target shut off time in s. Since the article does not mention that any participants forget to shut off the movie, it is assumed that all did.

**Table 7:** Confounded Age Contrasts by ProM Subdomain (Vigilance, ProM Proper, Habitual ProM) and Cue Type (Event, Time) in Laboratory Settings.

First Author & Year	Exp. no.	Condition	Ongoing Task	No. cues	# Cue-Action pairs	Lenient/Strict Scoring	Young n	Older n	ProM Young M	ProM Older M	ProM Age Effect	Confounds
**EC ProMP**												
Huppert '00 [52]	1	name & address	u/t	1	1	S	2992	191	0.68	0.20	-	dem
Mantyla '97 [61]	1	signature	u/t	1	1	S	500	500	0.54	0.30	-	dem
Cherry '01 [17]	1	specific cue	E&M STM	3	1	S	16	16	0.90	0.50	-	o,i
Cherry '01 [17]	1	general cue	E&M STM	3	1	S	16	16	0.54	0.29	-	o,i
Cherry '01 [17]	2	specific cue	E&M STM	3	1	S	20	20	0.53	0.62	+	o,i
Cherry '01 [17]	2	general cue	E&M STM	3	1	S	20	20	0.43	0.27	-	o,i
Cherry '01 [17]	3	specific/typical	E&M STM	3	1	S	12	12	0.86	0.61	-	o,i
Cherry '01 [17]	3	general/typical	E&M STM	3	1	S	12	12	0.67	0.44	-	o,i
Cherry '01 [17]	3	specific/atypical	E&M STM	3	1	S	12	12	0.78	0.75	-	o,i
Cherry '01 [17]	3	general/atypical	E&M STM	3	1	S	12	12	0.44	0.28	-	o,i
Cherry '03 [58]	1	low com./low sup./trial 1	E&M STM	3	1	S	18	18	0.28	0.67	+	o,i
Cherry '03 [58]	1	low com./low sup./trial 2	E&M STM	3	1	S	18	18	0.61	0.44	-	o,i
Cherry '03 [58]	1	low com./low sup./trial 3	E&M STM	3	1	S	18	18	0.72	0.67	-	o,i
Cherry '03 [58]	1	low com./high sup./trial 1	E&M STM	3	1	S	18	18	0.39	0.44	+	o,i
Cherry '03 [58]	1	low com./high sup./trial 2	E&M STM	3	1	S	18	18	0.50	0.61	+	o,i
Cherry '03 [58]	1	low com./high sup./trial 3	E&M STM	3	1	S	18	18	0.67	0.61	-	o,i
Cherry '03 [58]	1	high com./low sup./trial 1	E&M STM	3	3	S	18	18	0.22	0.22	=	o,i
Cherry '03 [58]	1	high com./low sup./trial 2	E&M STM	3	3	S	18	18	0.22	0.28	+	o,i
Cherry '03 [58]	1	high com./low sup./trial 3	E&M STM	3	3	S	18	18	0.22	0.17	-	o,i
Cherry '03 [58]	1	high com./high sup./trial 1	E&M STM	3	3	S	18	18	0.44	0.44	=	o,i
Cherry '03 [58]	1	high com./high sup./trial 2	E&M STM	3	3	S	18	18	0.56	0.22	-	o,i
Cherry '03 [58]	1	high com./high sup./trial 3	E&M STM	3	3	S	18	18	0.72	0.22	-	o,i
Einstein '90 [4]	1	no aid	E&M STM	3	1	S	12	12	0.47	0.47	=	o,i
Einstein '90 [4]	1	aid	E&M STM	3	1	S	12	12	0.83	0.69	-	o,i
Einstein '90 [4]	2	familiar	E&M STM	3	1	S	12	12	0.28	0.36	+	o,i
Einstein '90 [4]	2	unfamiliar	E&M STM	3	1	S	12	12	0.83	0.94	+	o,i
Einstein '92 [8]	1	1 trg/short	E&M STM	3	1	S	12	12	0.58	0.53	-	o
Einstein '92 [8]	1	1 trg/long	E&M STM	3	1	S	12	12	0.42	0.61	+	o
Einstein '92 [8]	1	4 trg/short	E&M STM	3	4	S	12	12	0.58	0.19	-	o
Einstein '92 [8]	1	4 trg/long	E&M STM	3	4	S	12	12	0.47	0.11	-	o
Einstein '92 [8]	2	4 trg	E&M STM	3	4	S	12	12	0.53	0.14	-	o
Einstein '95 [55]	3	q&a	Q&A	6	1	S	18	13	0.93	0.86	-	o
McDaniel '03 [5]	2b	full	paragraphs	8	2	S	12	12	0.97	0.93	-	o
McDaniel '03 [5]	2b	divided	paragraphs	8	2	S	12	12	0.87	0.87	=	o
McDaniel '03 [5]	1	5 s/unfilled	paragraphs	8	2	S	20	20	0.90	0.45	-	o
McDaniel '03 [5]	1	5 s/filled	paragraphs	8	2	S	20	20	0.85	0.35	-	o
McDaniel '03 [5]	1	15 s/unfilled	paragraphs	8	2	S	20	20	0.85	0.48	-	o
McDaniel '03 [5]	1	15 s/filled	paragraphs	8	2	S	20	20	0.82	0.52	-	o
McDaniel '03 [5]	1	5 s/unfilled/rehearsal	paragraphs	8	2	S	20	20	0.90	0.74	-	o
McDaniel '03 [5]	1	5 s/filled/rehearsal	paragraphs	8	2	S	20	20	0.85	0.47	-	o
McDaniel '03 [5]	1	15 s/unfilled/rehearsal	paragraphs	8	2	S	20	20	0.85	0.60	-	o
McDaniel '03 [5]	1	15 s/filled/rehearsal	paragraphs	8	2	S	20	20	0.82	0.57	-	o
McDaniel '03 [5]	2a	break/full	paragraphs	8	2	S	40	40	0.93	0.79	-	o
McDaniel '03 [5]	2a	break/divided	paragraphs	8	2	S	40	40	0.78	0.52	-	o
McDaniel '03 [5]	2a	trivia/full	paragraphs	8	2	S	40	40	0.82	0.53	-	o
McDaniel '03 [5]	2a	trivia/divided	paragraphs	8	2	S	40	40	0.77	0.40	-	o
Cherry '99 [56]	1	low IQ	E&M STM	6	1	S	24	24	0.65	0.40	-	o,i
Cherry '99 [56]	1	high IQ	E&M STM	6	1	S	24	24	0.68	0.69	+	o,i
Reese '02 [57]	1	low IQ	E&M STM	6	1	S	32	32	0.59	0.51	-	o,i
Reese '02 [57]	1	high IQ	E&M STM	6	1	S	32	32	0.64	0.65	+	o,i
Cockburn '94 [62]	1	RBMT	u/t	0	0	L	44	43	0.87	0.81	-	item
Kidder '97 [18]	1	DOW/ProM	u/t	5	1	L	90	80	0.45	0.25	-	item, e(6y,23o)
Kliegel '00 [63]	1	RBMT	u/t	1	1	S	31	31	0.48	0.60	+	item
Martin '03 [40]	1	RBMT	u/t	1	1	S	40	40	0.63	0.83	+	item
**EC Vigilance**												
Bastin '02 [106]	1	12-event/recall absent	WMLVar	12	1	S	24	24	1.00	0.99	-	o
Bastin '02 [106]	1	12-event/recall present	WMLVar	12	1	S	24	24	0.95	0.93	-	o
Bastin '02 [106]	1	6-event/recall absent	WMLVar	6	1	S	24	24	0.99	1.00	+	o
Bastin '02 [106]	1	6-event/recall present	WMLVar	6	1	S	24	24	0.84	0.79	-	o
Einstein '00 [4]	1	no del/standard	paragraphs	8	2	S	20	20	0.97	0.95	-	o
Einstein '00 [4]	1	no del/divided	paragraphs	8	2	S	20	20	0.96	0.88	-	o
Einstein '00 [4]	1	delay exe/standard	paragraphs	8	2	S	20	20	0.82	0.77	-	o
Einstein '00 [4]	1	delay exe/divided	paragraphs	8	2	S	20	20	0.72	0.48	-	o
Einstein '00 [4]	2	10s/unfilled	paragraphs	4	2	S	24	24	0.88	0.42	-	o
Einstein '00 [4]	2	10s/filled	paragraphs	4	2	S	24	24	0.75	0.42	-	o
Einstein '00 [4]	2	30s/unfilled	paragraphs	4	2	S	24	24	0.88	0.44	-	o
Einstein '00 [4]	2	30s/filled	paragraphs	4	2	S	24	24	0.79	0.55	-	o
**TC ProMP**												
Einstein '95 [55]	3	q&a	Q&A	6	1	S	18	13	0.65	0.32	-	o
**TC Vigilance**												
Bastin '02 [106]	1	high freq./recall absent	WMLVar	12	1	S	24	24	0.94	0.88	-	o
Bastin '02 [106]	1	high freq./recall present	WMLVar	12	1	S	24	24	0.87	0.57	-	o
Bastin '02 [106]	1	low freq./recall absent	WMLVar	6	1	S	24	24	0.94	0.72	-	o
Bastin '02 [106]	1	low freq./recall present	WMLVar	6	1	S	24	24	0.80	0.48	-	o

*Note.* Confounds: o  =  ongoing task was easier for older adults; i  =  older adults were substantially more intelligent than younger adults; dem  =  older group had higher proportion of participants who scored in dementia range on screening tests; e(6y, 23o)  =  exclusion of subjects (6 young, 23 old) for various reasons; ep (0y,5o)  =  exclusion of subjects (0 young, 5 old) because of low ProM performance; item  =  participants were to request a personal item back but the items varied from participant to participant; #cues  =  number of ProM cues varied from participant to participant.

Ongoing task: u/t  =  unrelated tasks; Q&A  =  questions and answers; PA  =  paired associates; WM  =  working memory; E&M STM  =  Einstein & McDaniel Short Term Memory task (WM task); WML3  =  working memory task; WMLVar  =  working memory task.

a Patton'93: ProM task was “to shut off the movie after exactly 30 min had elapsed”. However, the article reports only deviation from target shut off time in s. Since the article does not mention that any participants forget to shut off the movie, it is assumed that all did.

### Characteristics of Age Contrasts

The search yielded 162 contrasts free of age-related confounds and 71 contrasts with age confounds. Figure 5 shows the number of unconfounded (black filled bar sections) and confounded (gray filled bar sections) age contrasts by prospective memory subdomain, cue type, and study type (Panels 5a through 5d). This highlights that there are only a few studies that have investigated prospective memory proper without confounding age with other variables such as participants' intelligence or ease of the ongoing task. Moreover, almost all of the studies investigating event-cued prospective memory proper did so in laboratory settings whereas almost all of the studies investigating time-cued prospective memory proper did so in naturalistic settings. Thus, the scarcity of data makes it impossible to directly compare, for example, age-related declines in event-cued versus time-cued prospective memory proper under laboratory versus naturalistic conditions. Similarly, there have been no laboratory studies of habitual prospective memory and only one study of event-cued habitual prospective memory in a naturalistic setting. Finally, Figure 5 underscores that the majority of previous research conducted under the umbrella of prospective memory has investigated vigilance rather than prospective memory proper. Most importantly, Figure 5 highlights that age-related effects in prospective memory performance for most cells formed by crossing subdomain, cue type, and study type have yet to be investigated and cautions against making meta-analytic conclusions about any contrast that is confounded with some other contrast, for example, age declines on laboratory versus naturalistic tasks because such comparisons at this time are confounded with type of prospective memory cue. Figure 5 also highlights that a substantial number of age contrasts are confounded by other variables, with the majority of the confounds likely to minimize age-related differences (i.e., intelligence and ongoing task difficulty confounds). In turn, the data in Figure 5 cast doubt on the conclusions of the Henry et al. meta-analysis, as they did not take the above considerations into account.

**Figure 5:** Panels 1a through 1d show the number of unconfounded (black filled bar sections) and confounded (gray filled bar sections) age contrasts by ProM subdomain, cue type, and study type. Panels 5e and 5f show the distribution of sample sizes for laboratory versus naturalistic studies.

Figures 5e and 5f show the distribution of group sample sizes for laboratory versus naturalistic studies. This shows that the number of participants in the vast majority of previous studies was so small that these studies did not have sufficient statistical power to discover even effect sizes as large as 1 *SD*. In turn, this lack of statistical power may alone produce a “substantial number” of studies showing no age decline in prospective memory even if age declines in prospective memory are large, even if they are larger than age declines in retrospective memory as argued by Craik [2], [3]. It is a well known fact that outcomes of underpowered studies cannot be used to argue for the existence of null findings.

### Aging and Prospective Memory

#### Meta-Analysis via Visualization and Modelling

Figure 6 shows the size of raw age declines as a function of older adults' performance for event-cued prospective memory proper, event-cued vigilance and time-cued vigilance tested in the laboratory, and for time-cued prospective memory proper and time-cued habitual prospective memory tested in natural settings. It also includes the best fitting estimated *d* derived by double variate square error minimization methods and associated nonparametric 95% confidence intervals derived by bootstrapping using 10,000 samples [47]–[49]. The figure highlights that the majority of all contrasts reveal age-related declines in prospective memory measured in the laboratory and that such age declines depend on prospective memory subdomain–they are largest for event-cued prospective memory proper (the best fitting *d* = −1.13) and smallest for event-cued vigilance (the best fitting *d* = −.77). Specifically, the age declines on event-cued prospective memory proper are larger than on event-cued vigilance (*d* difference = −0.36 with bootstrap 95% *CI* = (−0.60,−0.08)). In contrast, the majority of all age contrasts showed substantial age improvements in natural settings (the best fitting *d* = 0.53 for time-cued prospective memory proper and 0.76 for time-cued habitual prospective memory).

**Figure 6:** The figure shows younger adults performance as a function of older adults' performance for event cued (EC) prospective memory proper, EC vigilance and time cued (TC) vigilance tested in the laboratory, and for TC prospective memory proper and TC habitual prospective memory tested in natural settings. The figure also includes the best fitting estimated d derived by double variate square error minimization methods and bootstrap 95% confidence intervals. The figure highlights that the majority of all contrasts reveal age-related declines in ProM measured in the laboratory and that such age declines depend on ProM subdomain–they are largest for EC prospective memory proper (the best fitting *d* = −1.13) and smallest for EC vigilance (the best fitting *d* = −.77). In contrast, the majority of all age contrasts showed substantial age improvements in natural settings (the best fitting *d* = 0.53 for TC prospective memory proper and 0.76 for TC habitual prospective memory). Importantly, the figure highlights that the size of raw age-related differences in individual studies is determined by the degree of ceiling effects, that is, the distance of the lower scoring group from the maximum achievable score. The bottom right panel summarizes the findings; it depicts a summary graph of the average effect sizes by ProM subdomain, cue type, and task type. It highlights that under controlled laboratory conditions all subdomains of ProM for which sufficient data exist show substantial age-related declines, and more importantly, that such age declines are much larger for EC prospective memory proper (d = −1.13) than for EC vigilance (d = −0.77). In contrast, under naturalistic conditions, older adults perform better than younger adults on ProM tasks that have been investigated: TC prospective memory proper (0.53) and TC habitual prospective memory (0.76).

Importantly, this figure highlights that the size of raw age-related differences in individual studies is determined by the degree of ceiling effects, that is, the distance of the lower scoring group from the maximum achievable score. Accordingly, these ceiling limited scores obscure the magnitude of true age-related differences in prospective memory performance and underscore that any meta-analysis that estimates *d* by using parametric information (e.g., *d_p_* or *d_phi_* calculated from means, standard deviations, *r*s, *t*s, *F*s, etc. reported in Henry et al. [14]) severely underestimates the size of true effects [15], [16].

The findings are summarized in Figure 6, bottom right panel, depicting a summary graph of the average effect sizes by prospective memory subdomain, cue type, and task type. It highlights that under controlled laboratory conditions all subdomains of prospective memory for which sufficient data exist show substantial age-related declines, and more importantly, that such age declines are much larger for event-cued prospective memory proper (*d* = −1.13) than for event-cued vigilance (*d* = −0.77) (*d* difference = −0.36, bootstrap 95% *CI* = (−0.60,−0.08)). Moreover, age declines are also larger on time-cued vigilance (*d* = −0.95) than event-cued vigilance (*d* = −0.77) but this difference failed to reach statistical significance (*d* difference = −0.18, bootstrap 95% *CI* = (−0.47,0.03)). Unfortunately, a similar comparison for the prospective memory proper subdomain is impossible due to insufficient data. In contrast, under naturalistic conditions, older adults perform better than younger adults on prospective memory tasks that have been investigated: time-cued prospective memory proper (*d* = 0.53) and time-cued habitual prospective memory (*d* = 0.76) and age improvements appear larger on time-cued habitual prospective memory versus time-cued prospective memory proper but this difference failed to reach significance (*d* difference = −0.23, bootstrap 95% *CI* = (0.51,0.02)). Finally, it is impossible to directly compare age declines in laboratory versus naturalistic settings as the subdomain/cue type combinations studied in naturalistic settings have not been studied in the laboratory and vice versa.

#### Meta-Analysis via Robust Techniques

Table 8 shows a summary of the meta-analysis for all outcomes (i.e., a participant may have contributed data to more than one condition/age-contrast) and for independent outcomes only (i.e., each participant contributed data to only one condition/age-contrast). For each task type, subdomain, and cue type, it shows the number of age-contrasts available (*k*) and a summary of the outcomes–number of age contrasts showing age decline, age parity (i.e., no differences), and age improvement in prospective memory– and *d_probit_* and, for the independent outcomes only, binomial probability that each outcome is due to chance alone rather than due to age-related influences. To illustrate, for event-cued prospective memory proper, considering all outcomes, the table shows that 18 age contrasts showed age declines, no age contrast showed parity, and no age contrast showed age improvement. Considering only the independent outcomes, the table shows that 13 age contrasts showed age declines, no age contrast showed parity, and no age contrast showed age improvement. In turn, this result is associated with binomial *p*<0.001. Accordingly, these data suggest that event-cued prospective memory proper declines with aging. In summary, the binomial test confirmed what is readily apparent from the graphical summaries of the data: statistically significant age-related declines were observed in all laboratory conditions for which there is enough data available to conduct statistical testing: event-cued prospective memory proper, event-cued vigilance, and time-cued vigilance. Similarly, binomial tests confirmed that statistically significant age-related improvements were found in all natural setting conditions for which the data are available: time-cued prospective memory proper and time-cued habitual prospective memory.

**Table 8:** Summary of Meta-Analysis.

	All Outcomes				Independent Outcomes				
	K		De-Eq-Im	d_probit_	K	N	De-Eq-Im	*p*	d_probit_
**AGE CONTRASTS WITH NO CONFOUNDS**									
**LABORATORY**									
**Prospective Memory Proper (ProMP)**									
Event Cued	18		18-0-0	−0.99	13	1528	13-0-0	<.001	−0.96 (−1.22,−0.69)
Time Cued	1		1-0-0	–	1		1-0-0	–	Insufficient data
**Vigilance**									
Event Cued	94		88-3-4	−0.71	48	2200	44-2-2	<.001	−0.61 (−0.73,−0.49)
Time Cued	19		15-3-1	−0.79	17	738	13-3-1	.002	−0.82 (−1.08,−0.56)
**Habitual Prospective Memory (HProM)**									
Event Cued	0		0-0-0	–	0				No data available
Time Cued	0		0-0-0	–	0				No data available
**NATURAL**									
**Prospective Memory Proper (ProMP)**									
Event Cued	2		1-0-1	–	2		1-0-1	–	Insufficient data
Time Cued	12		0-0-12	0.53	10	682	0-0-10	.002	0.54 (0.32,0.76)
**Vigilance**									
Event Cued	0		0-0-0	–	0				No data available
Time Cued	0		0-0-0	–	0				No data available
**Habitual Prospective Memory(HProM)**									
Event Cued	1		0-0-1	–			0-0-1	–	Insufficient data
Time Cued	15		0-0-15	0.77	15	574	0-0-15	<.001	0.78 (0.54,1.04)
**AGE CONTRASTS WITH AGE CONFOUNDS (all in laboratory)**									
**Favoring Old**									
ProMP, Event-cued	48		34-4-10	−0.45	30	1039	19-3-8	.052	−0.30 (−0.50,−0.10)
W/o delayed exe	36		22-4-10	−0.24	27	879	16-3-8	.015	−0.22 (−0.42,−0.02)
Delayed exe only	12		12-0-0	−0.91	3		3-0-0	–	Insuficient data)
ProMP, Time-cued	1		1-0-0	–	1		1-0-0	–	Insufficent data
Vigilance, Event-c.	12		11-0-1	−0.68	5	224	5-0-0	.063	−0.63 (−1.09,−0.17)
W/o delayed exe	6		5-0-1	−0.24	3		3-0-0	−	Insuficient. data
Delayed exe only	6		6-0-0	−0.85	2		2-0-0	−	Insuficient data
Time-cued vigilance	4		4-0-0	–	2		2-0-0	–	Insufficient data
**Favoring Young**									
ProMP, Event-cued	2		2-0-0	–	2		2-0-0	–	Insufficient data
**Unknown Effect**									
ProMP, Event-cued	4		2-0-2	–	4		2-0-2	–	Insufficient data

Note: De = decline, Eq = equal, Im = improvement. – = insufficient data

#### Conventional Meta-Analysis Using d_probit_ Effect Size Indices

To analyze these ceiling-limited data, the random effects model [44], [66] with *d_probit_* effect size indices was chosen rather than frequently used *d_p_* and *d_phi_* effect size indices because it is more appropriate for dichotomous data and because it yields less biased estimates of d across a much wider range of test sensitivities and is much less influenced by ceiling-limited scores (see above).

Table 8 shows the mean effect size indices and associated 99% confidence intervals for *d_probit_*. The mean effect sizes are similar to those derived via graphical and minimization modeling methods, although as expected due to the ceiling-limited nature of primary data, they are generally slightly smaller. Critically, age-related declines are larger on event-cued prospective memory proper than on event-cued vigilance, *p*<0.05. Age-related declines appear larger on time-cued vigilance than on event-cued vigilance in laboratory settings but the difference fell short of statistical significance. Similarly, age improvements appear to be larger on time-cued habitual prospective memory than on time-cued prospective memory proper in natural settings but this difference also fell short of statistical significance due to the small number of studies.

Figure 7 highlights deleterious effects of ceiling effects on commonly used effect size *d_p_* using both Henry et al. [14] data set and much larger data set included in the present study. Panel A shows *d_p_* calculated by Henry et al. as a function of older adults performance (test difficulty) for laboratory conditions that were free of age-confounds only (color of the circles indicate prospective memory subdomain: red = event-cued prospective memory proper, blue = event-cued vigilance, green = time-cued vigilance). As expected from the modeling work (see Figure 4 and Table 2), Panel A highlights that the size of age declines measured by effect size index *d_p_* decreases as performance of older adults increases, as the test becomes easier and data are more afflicted by ceiling effects. Panel B demonstrates this deleterious effect of ceiling effects on *d_p_* using much larger data set identified for the current study. Panel C highlights that even age declines measured by *d_probit_* are dependent on the test difficulty but, consistent with previous simulations [43], less so. Finally, Panel D highlights that *d_p_* underestimates the size of age decline relative to *d_probit_*; age declines measured by *d_p_* are smaller then age declines measured by *d_probit_*. Thus, these graphical presentations may help a traditional meta-analysist to identify the fundamental problems with the primary data as well as with the selection of effect size indexes [67] and perhaps encourage search for alternative approaches to meta-analysis.

**Figure 7:** Figure highlights deleterious effects of ceiling effects on commonly used effect size *d_p_* using both Henry et al. [14] data set and much larger data set included in the present study. Panel A shows *d_p_* calculated by Henry et al. [14] as a function of older adults performance (test difficulty) for laboratory conditions that were free of age-confounds only (color of the circles indicate prospective memory subdomain: red = event-cued prospective memory proper, blue = event-cued vigilance, green = time-cued vigilance). Panel A highlights that the size of age declines measured by effect size index *d_p_* decreases as performance of older adults increases, as the test becomes easier and data are more afflicted by ceiling effects. Panel B demonstrates this deleterious effect of ceiling effects on *d_p_* using much larger data set identified for the current study. Panel C highlights that even age declines measured by *d_probit_* are dependent on the test difficulty but, consistent with previous simulations [43], less so. Finally, Panel D highlights that *d_p_* underestimates the size of age decline relative to *d_probit_*; age declines measured by *d_p_* are smaller then age declines measured by *d_probit_*.

#### Pattern of Age Decline Across the Adult Lifespan

What is the pattern of age-related declines or increases for various subdomains of prospective memory? Are such age declines linear across the adult lifespan? Or are age declines curvilinear showing no age-related changes until about 60 years of age followed by age-related declines? Figure 8 shows the results of a few studies that included more than two age groups, and thus, may allow us to gain some insight into the pattern of age-related declines for each prospective memory subdomain for which we have at least some data. Figure 8a shows performance on event cued prospective memory proper assessed using dichotomous measures in laboratory settings for several studies free of age-related confounds (C'07 = Cuttler & Graf [51], Q = questionnaire task, P = plug in phone task; D'87 = Dobbs & Rule [38]; S'04 = Salthouse, Berish, & Siedlecki [50]; U'01 = Uttl et al. [11], N = name task, L = letter task, C = envelope task; Z = Zimmerman & Meier [68]) and two population-based studies where age was confounded with increased occurrence of dementia (M'97 = Mantyla & Nilsson [61]; H'00 = Huppert, Johnson, & Nickson [52]). The unconfounded data clearly show that there is linear decline in event-cued prospective memory proper after about 65–70 years of age. Although the C'07/Q (Cuttler and Graf [51], questionnaire task), D'87 (Dobbs & Rule [38]), S'04 (Salthouse et al. [50]) and Z'05 (Zimmerman and Meier [68]) data show no or only minimal age declines between 25 and 65 years of age, these data are not interpretable because they are limited by ceiling effects, and thus, younger adults were unable to demonstrate better prospective memory. Figure 8b shows performance on event cued prospective memory proper assessed using two continuous measures (visual and auditory) in laboratory settings. The data are not limited by ceiling or floor effects and suggest that there are no or only minimal changes in EC prospective memory proper from approximately 20 to 60 years of age followed by age-related declines. Figure 8c shows performance on event-cued vigilance assessed using dichotomous measures in laboratory settings from a single study by Salthouse et al. [50]. Similar to the event cued prospective memory proper dichotomous data, the vigilance data for younger age groups (i.e., 20 to 70 years of age) are not interpretable because of ceiling effects, but the data for older adults (over 70 years of age) show age-related declines. Finally, Figure 8d shows performance on time cued prospective memory proper and on event cued prospective memory proper assessed in natural settings. The C'07 (Cuttler & Graf [51], conference call task) and L'90 (time cued; Levy & Clark [69]) data show performance increases with aging whereas the D'87 (event cued; Dobbs & Rule [38]) data show performance decreases with aging.

**Figure 8:** The pattern of age declines and improvements across the adult lifespan. Panel A shows performance on event cued prospective memory proper assessed using dichotomous measures in laboratory settings for three studies free of age-related confounds (in green: D'87 = Dobbs & Rule [38]; in dark green: S'04 = Salthouse et al. [50]; in blue: U'01 = Uttl et al. [11], N = name task, L = letter task, C = envelope task) and two population-based studies where age was confounded with increased occurrence of dementia (in orange: M'97 = Mantyla & Nilsson [61]; in purple: H'00 = Huppert, Johnson, & Nickson [52]). The D'87 and S'04 data are not interpretable for younger adults due to severe ceiling effects but the data from all studies show clear age-related declines for adults older than 60–70 years. Panel B shows performance on event-cued prospective memory proper assessed using two continuous measures (visual in red and auditory in blue) in laboratory settings. The data are not limited by ceiling or floor effects and suggest that there are no or only minimal changes in EC prospective memory proper from approximately 20 to 60 years of age followed by age-related declines. Panel C shows performance on event-cued vigilance assessed using dichotomous measures in laboratory settings from a single study by Salthouse et al. [50]. Similarly to the EC prospective memory proper dichotomous data, the vigilance data for younger age groups (i.e., 20 to 70 years of age) are not interpretable because of the ceiling effects but the data for older adults (over 70 years of age) show age-related declines. Panel D shows performance on time cued prospective memory proper (red) and on event cued prospective memory proper assessed in natural settings (blue). The L'90 (TC; Levy & Clark [69]) data show performance increases with aging whereas the D'87 (EC; Dobbs & Rule [38]) data show performance decreases with aging.

The data in Figure 8d highlight that the conclusions that older adults' prospective memory proper improves with age in natural settings but declines with age in laboratory settings [14] is premature. First, this conclusion is based on analyses that disregarded the distinction between event-cued and time-cued prospective memory and mixed many time-cued studies with a single or a few event-cued studies (see Figure 5) as if the type of cue could not affect performance. Second, the one unconfounded event-cued prospecive memory proper study in a natural setting that has been published [38] revealed age declines rather than age improvements.

In summary, the evidence regarding the pattern of age-related declines or improvements across the adult life span is very limited. However, the available evidence suggests that event-cued prospective memory proper assessed in the laboratory does not change until about 60 years of age and declines thereafter (see Figure 8b).

### Other Moderator Variables

#### Focal versus Non-Focal Cues

McDaniel and Einstein [6] argue that there are no age-related declines on prospective memory task for “focal” ProM cues, that is, “the features of the target cue that have been associated with the prospective memory intention are features that are processed because of the ongoing activity.” However, the data presented in support of their claim were confounded by severe ceiling effects: the younger adults' mean was 90% whereas the older adults' mean was 78% in the focal condition. As demonstrated by Figure 4f it is nearly impossible to detect even large (i.e., *d* = 1.0 standard deviation) age effects with this level of performance using dichotomous performance indices. Moreover, other studies of event-cued prospective memory proper where ProM cues were “focal” by McDaniel and Einstein's definition show robust age declines (e.g., [11], [38], [50]). Accordingly, at present, there is no evidence that aging does not affect prospective memory proper when prospective memory proper cues are “focal”.

This conclusion is firmly buttressed by the analysis of data recently extracted and classified as focal versus non-focal by McDaniel and Einstein themselves ([6], Table 7.4, p. 143–156). McDaniel and Einstein tabulated 82 age contrasts from event cued laboratory experiments irrespective of ceiling effects, age confounds, and ProM subdomains; classified each contrast as arising from the use of “focal”, “nonfocal”, or “indeterminate” ProM cues; but, surprisingly, did not attempt to statistically determine the strength of evidence for or against their claim that age declines are absent with focal ProM cues. Accordingly, Figure 9 shows the graphical analysis of the data reported in McDaniel and Einstein's Table 7.4; it shows the performance of older adults plotted against the performance of younger adults, for focal and non-focal ProM cues. The figure includes *d*s derived by modeling methods described above and 95% confidence intervals derived by bootstrapping methods. The circles indicate contrasts free of age confounds (i.e., ongoing task and intelligence confound) and squares indicate contrasts with ongoing task, intelligence, or both confounds.

**Figure 9:** The graphical analysis of the data reported in McDaniel and Einstein's Table 7.4 (p. 143–156) [6]; it shows performance of older adults plotted against performance of younger adults, for focal and non-focal ProM cues. The figure includes *d*s derived by graphical modeling methods including 95% confidence intervals derived by bootstrapping methods. The blue circles indicate contrasts free of age confounds (i.e., ongoing task and intelligence confound) and red squares indicate contrasts with ongoing task, intelligence, or both confounds favoring older adults. The figure highlights substantial age-related declines in ProM with both focal and non-focal cues even for this very selective and biased sample (see text for the explanation) of previously published data reported by McDaniel and Einstein [6], lending no support to their claims that aging does not affect prospective memory.

The data in Figure 9 lend no support to the claim that aging does not affect prospective memory–indeed they are evidence to the contrary. First, the simple, robust, ceiling effects resistant count methods show that (a) for focal cues, there are 27 age declines, and 6 age improvements (all except one arising from studies that confounded age with ease of the ongoing task, intelligence, or both), revealing significant age decline, *p* = 0.006, and (b) for non-focal cues, there are 36 age declines, and 3 age improvements, also indicating an overall age decline, *p*<0.001. Second, graphical modeling methods combined with bootstrapping methods show substantial age declines for both focal and non focal cues, *d_focal_* = −0.50 and *d_nonfocal_* = −0.72, respectively.

More importantly, the data presented by McDaniel and Einstein in Table 7.4 and shown in Figure 9 are biased towards minimizing age differences for a number of reasons. First, McDaniel and Einstein Table 7.4 omitted over 50% of all laboratory event-cued age contrasts identified in this review, and, even more importantly, it failed to include all unconfounded age contrasts of event-cued prospective memory proper listed in the first section of Table 3 (e.g., [11], [12], [38], [50], [70]) with the exception of Tombaugh et al. [29]. Thus, the data in McDaniel and Einstein's Table 7.4 and Figure 8 paint a very biased picture of age declines in ProM because, with the exception of Tombaugh et al. data, the table includes only event-cued prospective memory proper age contrasts where age confounds minimized age differences and event-cued vigilance age contrasts where age differences are much smaller than on event-cued prospective memory proper (this review's result). Second, Figure 9 highlights that there is substantial heterogeneity in the studies lumped together by Einstein and McDaniel. To illustrate, whereas many of the studies with focal cues confounded age with intelligence and ongoing task ease (always favoring older adults), only a few studies with non-focal cues have done so. Third, Figure 9 also highlights that a large number of studies were limited by severe ceiling effects that artificially minimize age differences and render any calculations of effect sizes based on *d_p_, d_phi_*, or even simple differences between mean proportions, meaningless (see [6]).

In summary, neither the current comprehensive meta-analysis nor the analysis of Einstein and McDaniel's [6] selective review of previously published data support the notion that age declines are absent with focal ProM cues. To the contrary, analyses of Einstein and McDaniel's data show that there are large robust age declines with both focal and non-focal cues even though many studies included in the analyses made the ongoing task easier for older adults (e.g., [4], [8], [17], [56]), compared very intelligent older adults with not so intelligent younger adults (e.g., [4], [17], [56]), left out more than 50% of published research, and left out all but one age contrast of event-cued prospective memory proper.

#### Delayed Execution or ProM Task Chaining

In several experiments, Einstein, McDaniel, and their colleagues [5], [71] chained two prospective memory tasks by asking participants to not respond to a ProM cue until some other cue arrives. Because only a few experiments used this ProM task chaining, the available data are insufficient for a meaningful meta-analysis. However, consistent with theoretical expectation, the existing data suggest that chaining ProM tasks results in larger prospective memory declines on chained tasks than on a single ProM tasks.

### Effects of Age Confounds

Table 8 also provides information about the age-confounded studies. For each study type, prospective memory subdomain, and cue type, the table lists the number of contrasts (k); the number of studies showing age decline, age parity, and age improvement (e.g., 15-1-0); and *d_probit_* for all contrasts as well as for a subset of independent contrasts.

#### Ease of Ongoing Task

As expected, age differences were reduced when the ongoing task was made easier for older adults than for younger adults. This conclusion is supported both by graphical analysis as well as by probit based effect size indices (see Table 8). In turn, these results suggest that both prospective memory proper and vigilance are resource-demanding rather than automatic and that age declines seen on prospective memory proper and vigilance are at least in part due to age declines in available processing resources as argued by Craik [2], [3].

One might argue that Einstein and McDaniel [4] and others who incorporated the ease of ongoing task confound into their designs aimed to equate functional difficulty of ongoing tasks for younger and older adults and that age declines under these “functionally equated” conditions reflect true age differences in prospective memory. However, it is misleading to interpret the results of these confounded studies as showing no or small age declines in prospective memory. First, far more sophisticated dual task designs will be necessary to establish functional equivalence of the ongoing task for younger and older adults beyond looking at equivalence of means in ongoing task performance. The lack of age differences in ongoing task performance may mean many different things, for example, the easy ongoing task for older adults required very few resources, and even though older adults allocated more of their resources to prospective memory task than younger adults they still managed to match younger adults performance because the ongoing task was designed to be easier for them. Second, close examination of the studies that attempted to functionally equate ongoing task difficulty suggests that equating of ongoing task demands is difficult, if not impossible even, in laboratory conditions. To illustrate, Einstein and McDaniel [4], who pioneered this procedure, aimed to equate ongoing task (working memory task) demands by presenting older versus younger adults with shorter word lists but their own analysis of actual ongoing task performance revealed that older adults significantly outperformed younger adults. Thus, the lack of statistically significant age differences in Einstein and McDaniel's [4] study can be interpreted only in light of this ease of ongoing task confound that did not succeed in equating performance on the ongoing task but made it easier for older versus younger adults. Third, it is impossible to equate ongoing task demands for younger and older adults in real-life, for example, by slowing down traffic for older adults and speeding it up for younger adults at the same time. Thus, the results of laboratory studies showing smaller age differences in prospective memory when younger adults are given a difficult ongoing task and older adults are given an easy ongoing task have no ecological validity and are merely an exercise in academic discourse.

The designs with ongoing task confounds can answer only one question: what are age differences in prospective memory *when these confounds are present*, that is, when the ongoing task is made easier for older versus younger adults? The answer provided by the present meta-analysis is that age declines remain substantial even after these attempts to “functionally equate” ongoing task demands. Moreover, by comparing the size of age declines on confounded and non-confounded studies, the present meta-analysis suggests that ongoing task demands influence older adults' performance on both vigilance and prospective memory proper, strongly suggesting that neither vigilance nor prospective memory proper retrieval is automatic contrary to some recent claims by Einstein, McDaniel and their colleagues [4], [7], [72].

#### Participants' Verbal Intelligence

Previous research has demonstrated that ProM is positively correlated with intelligence (e.g., [11], [56], [60]). In two studies, Cherry and her colleagues ([56], [57]) concluded that ProM is related to intelligence and that ProM does not decline with aging, consistent with McDaniel and Einstein's [72] multi-process framework. However, close inspection of the data and participants' characteristics reveals that Cherry and LeCompte [56] and Reese and Cherry [57] confounded intelligence with age–older adults scored 1.5 to 1.7 SDs higher on verbal intelligence tests than younger adults (this difference corresponds to a 22.5 to 25.5 IQ point difference). While older adults are expected to score higher on verbal intelligence tests than younger adults, the expected difference is much smaller, between 0.3 to 0.8 SD rather then 1.5 to 1.7 SD [73]–[76]. When younger and older groups with more comparable verbal intelligence scores are compared in these two studies (i.e., “high” intelligence young group and “low” intelligence older group), substantial age declines in ProM are apparent in both.

## Discussion

The meta-analysis of laboratory findings reveals a substantial body of evidence for the following key conclusions: First, both event-cued prospective memory proper and vigilance decline with aging. Second, age declines are much larger on prospective memory proper than on vigilance. And third, age declines in prospective memory proper (*d* = 1.13) are as large or even larger than those found with classical retrospective memory tests such as verbal learning free recall tests (*d* = 1.01, Spencer & Raz [23]; *d* = 0.97, La Voie & Light, 1994). The meta-analysis also suggests that age declines in prospective memory are generally small until the 50s or 60s and accelerate thereafter. In contrast, the meta-analysis of naturalistic findings indicates that for time-cued prospective memory proper and habitual prospective memory, the performance of older adults surpasses the performance of younger adults. Although only one study examined event-cued prospective memory proper in natural settings, its results suggest that naturalistic event-cued prospective memory proper may decline the same way as event-cued prospective memory proper assessed in the laboratory (see Figure 8d). Moreover, the meta-analysis reveals no evidence that aging spares any particular domain of ProM as argued by Einstein, McDaniel, and their colleagues (e.g., [4]–[6], [77]).

Importantly, the meta-analysis also reveals severe methodological problems with many previous studies of ProM: most significantly, severe ceiling effects that artificially reduce observed age differences (see Figures 1, 2, & 4; initially reported by Uttl [15], [16], and recently replicated by McDaniel & Einstein [6] on a small subsample of available data); small sample sizes that make it nearly impossible to find statistically significant age-related declines (see Figures 5e and 5f); failure to distinguish between subdomains of prospective memory, for example, between vigilance and prospective memory proper; and the presence of age-related confounds that reduce observed age differences. These methodological problems seem to be solely responsible for “a significant number of studies [that] show little or no age-related decrements in prospective memory performance” [5]. Indeed, all studies cited by McDaniel and Einstein [5] as showing no age-related declines in ProM are either: (a) studies of vigilance; (b) confounded by ease of ongoing task favoring older adults [4], [8], [17], [55]; (c) confounded by intelligence favoring older adults [4], [56], [57]; (d) suffering from severe ceiling effects [5], [55]; and/or (e) claiming no age declines based on sample sizes so small that even large age-related declines are undetectable (i.e., their statistical power is astonishingly small) [4]). In turn, “the puzzle of inconsistent age-related declines in prospective memory” (a book chapter title) [78] is shown to be an artifact of inadequate methodologies and conceptual confusions.

The meta-analysis is broadly consistent with Craik's claim [2], [3] that age declines in ProM are large and that the size of age declines varies with demands on processing resources. Specifically, age declines are larger for event-cued prospective memory proper than for event-cued vigilance, larger when the ongoing task is made more rather than less demanding for older adults, and they are larger for time-cued vigilance than for event-cued vigilance. Moreover, the evidence suggests that age declines on event-cued prospective memory proper (the most resource demanding of the three prospective memory subdomains) are at least as large as age-related declines on the most resource demanding retrospective memory task–free recall–if not larger. This latter conclusion is consistent with the results of a few studies that have examined age-related differences in prospective memory proper using continuous measures of similar high reliability as those used to investigate age-related differences in free recall [12].

The meta-analysis lends no support to claims that ProM is an exception to generally found age declines [4]. The meta-analysis also does not support the multi-process framework claiming that the retrieval of a previous plan is automatic when prospective memory cues are focal [6], [79]. First, the experimental results offered by McDaniel, Einstein, and their colleagues [6], [79] are unambiguously confounded by severe ceiling effects, and thus, uninterpretable. Second, a number of studies including those by Cuttler & Graf [51], Salthouse et al. [50], and Uttl et al. [11], used focal ProM cues and found substantial age declines in prospective memory proper. And third, the analysis of McDaniel and Einstein's [6] selective compilation of the data extracted from the published literature also reveals substantial age declines on both focal and non-focal ProM cue tasks, strongly contradicting the notion that aging spares prospective memory with focal cues (see Figure 9).

The finding that age declines on event-cued prospective memory proper are much larger than age declines on event-cued vigilance adds to a growing body of literature demonstrating dissociations between prospective memory proper and vigilance (e.g., [16], [21]) and highlights the need for conceptual clarity, for using appropriate labels that clearly denote what is measured and studied by a particular investigation [1]. In the absence of such labels, the field is in danger of simultaneously discussing and arguing about the properties of apples (prospective memory proper), oranges (vigilance), and occasionally, of bananas (habitual prospective memory).

As with experimental studies, meta-analysis depends critically on the methodology employed by meta-analysts, most critically, on identification of all relevant studies, assessment of each primary study quality and design features, selection of appropriate outcome measures and effect size indices, appropriate analysis of effect size indices, and equally importantly, on blocking studies by experimental design and quality. The comparison between the present and Henry et al. [14] meta-analysis highlights that disregarding these methodological considerations leads not only to unsupported conclusions but also prevents meta-analysts from identifying important trends and factors in the previous research. While Henry at al. [14] argued that age declines in prospective memory are generally smaller that those found in retrospective memory and even absent when ongoing task demands are minimal, the present meta-analysis demonstrates that that finding was an artifact of failure to include all relevant published studies; to consider reliability differences between prospective memory and retrospective memory measures; to consider widespread ceiling effects in primary data diminishing observed age differences; to consider the influence of prospective memory subdomain on size of age declines; to block primary studies by presence of age confounds reducing observed age declines in prospective memory; and to use effect size indices and meta-analytic methods appropriate for dichotomous outcome data. Moreover, attention to conceptual issues also revealed that the research in some domains of prospective memory is so scarce as to prevent any conclusions about the effects of aging on these subdomains of prospective memory at this time.

The key conclusions reached in this article are supported by outcomes of all three meta-analytic approaches: the robust count method, the graphical model fitting method, as well as more traditional meta-analysis based on d***_probit_*** effect size index that underestimates *d* less then *d_p_* or *d_phi_* indices [43]. However, the graphical meta-analysis combined with effect size model fitting has several advantages over the count and traditional method: it makes obvious many fundamental problems with primary data including ceiling effects and yields unbiased estimate of effect size largely unaffected by widespread ceiling effects and low reliability of prospective memory indices. One glance at the graphical plots of primary data shown in Figure 6 transparently informs the reader about both the ceiling effects afflicting primary data as well as the sizable age declines and improvements in various prospective memory subdomains and settings (see also Figure 8)

The current meta-analysis of the relationship between prospective memory and aging highlights the feature advantages of quantitative reviews over narrative reviews: the meta-analysis allows systematic, explicit, quantitative, and thus a more objective review of the literature, and is uniquely suitable for resolving disagreement between narrative reviews that frequently come to completely opposite conclusions. The present meta-analysis shows that there is no evidence for the claim that “prospective memory seems to be an exciting exception to typically found age-related decrements in memory.” [4]. Instead, it strongly supports the position that ProM declines with aging [1]–[3], [11] and that such age declines vary with the ProM subdomain [1], [11], experimental settings [13], [14], and resource demands [2], [3].
